# Modeling and Mathematical Analysis of the Dynamics of HPV in Cervical Epithelial Cells: Transient, Acute, Latency, and Chronic Infections

**DOI:** 10.1155/2022/8650071

**Published:** 2022-08-23

**Authors:** Juan Carlos Sierra-Rojas, Ramón Reyes-Carreto, Cruz Vargas-De-León, Jorge Fernando Camacho

**Affiliations:** ^1^Maestría en Matemáticas Aplicadas, Facultad de Matemáticas, Universidad Autónoma de Guerrero, 39087, Chilpancingo, Guerrero, Mexico; ^2^División de Investigación, Hospital Juárez de México, 07760 CDMX, Mexico; ^3^Maestría en Ciencias de la Complejidad, Universidad Autónoma de la Ciudad de México, 03100 CDMX, Mexico

## Abstract

The aim of this paper is to model the dynamics of the human papillomavirus (HPV) in cervical epithelial cells. We developed a mathematical model of the epithelial cellular dynamics of the stratified epithelium of three (basale, intermedium, and corneum) stratums that is based on three ordinary differential equations. We determine the biological condition for the existence of the epithelial cell homeostasis equilibrium, and we obtain the necessary and sufficient conditions for its global stability using the method of Lyapunov functions and a theorem on limiting systems. We have also developed a mathematical model based on seven ordinary differential equations that describes the dynamics of HPV infection. We calculated the basic reproductive number (*R*_0_) of the infection using the next-generation operator method. We determine the existence and the local stability of the equilibrium point of the cellular homeostasis of the epithelium. We then give a sufficient condition for the global asymptotic stability of the epithelial cell homeostasis equilibrium using the Lyapunov function method. We proved that this equilibrium point is nonhyperbolic when *R*_0_ = 1 and that in this case, the system presents a forward bifurcation, which shows the existence of an infected equilibrium point when *R*_0_ > 1. We also study the solutions numerically (i.e., viral kinetic *in silico*) when *R*_0_ > 1. Finally, local sensitivity index was calculated to assess the influence of different parameters on basic reproductive number. Our model reproduces the transient, acute, latent, and chronic infections that have been reported in studies of the natural history of HPV.

## 1. Introduction

Human papillomavirus (HPV) is small, nonenveloped, icosahedral DNA viruses that have a diameter of 52-55 nm. HPV is one of the most common sexually transmitted diseases in the world, and it is the principal causative agent of cervical cancer (CC), which occurs in 99.7% of cases [1]. This is a large family of small viruses that are classified into low- and high-risk (HR) genotypes and which can cause abnormal cell proliferation, manifesting from epithelial warts to high-grade cervical intraepithelial neoplasia (CIN) [2].

At the cellular level, HPV infects keratinocytes (i.e., cells that are the most predominant in the epidermis). Traditionally, the epidermis is segmented into distinct structural and functional compartments, which are called the cornified layer (stratum corneum), granular layer (stratum granulosum), spinous layer (stratum spinosum), and the deepest layer the basal layer (stratum basale) (see Figure 1). Keratinocytes differentiate as they move through the cell layers, starting as basal keratinocytes. The keratinocytes produce more and more keratin, and they eventually undergo natural cell death and detachment (anoikis). The cornified keratinocytes that form the outermost layer of the epidermis are constantly shed off and replaced by new cells [3]. The differentiation can be lateral and suprabasal: in the first, other cells of the same stratum are produced; and in the second, other cells that change stratum are produced [4]. When a cell is infected by HPV, it retains this capacity for cell differentiation.

The infection is produced by the exposure of the stratum basale cells together with a HPV particle when microtraumas occur in the epithelium during sexual activity [5, 6]. The virus only infects stratum basale cells because they contain the receptors that allow binding with the L1 protein in the capsid of the virus [7, 8].

During the process of infection by HR genotypes, there is no viremic phase, replication is nonlytic, and levels of viral gene expression are kept low in the basal epithelium. This limits the innate immune response and adaptive is delayed, which favors the establishment of viral infection. Furthermore, the E6 and E7 oncoproteins interfere with the activation levels of type I interferon in the infected cell, which prevents the initiation of intracellular antiviral responses [9, 10].

The HPV replicative cycle can last between 6 and 12 weeks, which considerably expands the viral genome. This results in new mature viral particles that can reach 1,000, which are released when rupture of the cell membrane occurs [11].

As illustrated in Figure 2, the release of viral loads from infected cells produces viral kinetics that allows us to classify the infection as transient, acute, latent, or chronic. The first is transient when viral genetic material is present in the host for a short period, and there is no infection in the cells of the stratum basale. The viral load is removed until its complete elimination during the following days. The second is acute when the infection is presented, replicates the viral genome, produces viral particles, and is eventually cleared. The third is latent when acute infections only appear to clear, but the viral genome remains in the infected cell without detectable activity. Finally, the fourth is chronic if genetic material is not eliminated during the acute infection but continues to increase the viral activity over time [12, 13].

The persistence of HR HPV infection is one of the principal causes of CIN I, II, or III and cancer. Although it is not clear whether the viral load has a causal effect on increasing the risk of cervical lesions and cancer in HPV-infected women, a high viral load is associated with the persistence of HPV infection. Thus, viral load may be a marker of HPV persistence [14].

A retrospective natural history study of HPV infections through serial HPV viral load measurement in 261 untreated women with type-specific HPV DNA detected has shown a regression or decrease of a clonal cell population HPV-infected when the infection was latent [13]. This indicates that the kinetics of viral load can illustrate predictive scenarios on regression or progression of the type of viral infection presented by a HR HPV [13]. A protocol for a cohort study, called PAPCLEAR, has recently been reported, which was aimed at better understanding the course and natural history of cervical HPV infections in healthy, unvaccinated, and vaccinated young women [15]. This study will be relevant because of its impact in the clinic thanks to the possible integration of longitudinal data to mathematical models.

A lot of literature has been published [16–20] on the mathematical modeling of viral infections, typically in human immunodeficiency virus, hepatitis B and C, and influenza. Although the literature reports studies on HPV modeling at the cellular level and viral kinetic scenarios [21–24], they do not show a direct relationship with the types of infection considering the different stratum of the squamous epithelium to show progression or regression of an infection by the HPV. Asih et al. [21] proposed a model that considers four compartments: susceptible cells, infected cells, precancerous cells, and cancer cells. They analyzed the local stability of the equilibrium points of the model and investigated the parameters that play an important role in the progression toward invasive cancer. Akimenko and Adi-Kusumo [22], and Sari and Adi-Kusumo [23] proposed two models of an age-structured subpopulations of susceptible, infected, precancerous, and cancer cells and unstructured subpopulation of HPV that aimed at gaining insight into the disease characteristics of cervical cancer. Verma et al. [24] developed a mathematical model of HIV/HPV coinfection of the oral mucosa. This model considered the cellular immune response and the basal and suprabasal layers of epithelial tissue but ignores viral transmission via suprabasal differentiation. They obtained simulations of the kinetics of an acute infection that tends to disappear over time and the kinetics of a chronic infection. Finally, Murall et al. [25] propose a viral dynamics model of the stratified epithelium of four layers. They simulated a scenario of a slow growing HR HPV infection that spontaneously regresses and another scenario where the infection is inoculated with few cells and the microabrasion repairs quickly. However, this mathematical model ignores the dynamics of the healthy stratified epithelium, and although it models the viral transmission via suprabasal differentiation, it does so with a linear term.

Motivated by the above, we propose a deterministic model that includes several layers of the healthy and infected squamous epithelium without the presence of the immune system to simulate *in silico* the types of infection reported in the literature when HPV infection occurs.

The structure of this manuscript is as follows. In Section 2, we will describe a model to epithelial cellular dynamics of healthy tissue, and we will study the stability of its equilibrium points. In Section 3, we will describe the dynamics of HPV in the stratified epithelium of the cervix, and we will calculate the basic reproductive number for the viral infection, its equilibrium points, and their corresponding local and global stabilities. Additionally, we will show that one of these equilibrium points, the infection-free equilibrium, can be nonhyperbolic and that in this case, there is a bifurcation; this result shows the existence of an infected equilibrium point.  Section 4 shows the typical values required in the model that describes the dynamics of HPV-infected tissue, and with them, it is estimated numerically the local bifurcation type that this model exhibits, the regions of existence and stability of its infected equilibrium point, and the simulation of different scenarios of interest that reproduce the transient, acute, latent, and chronic infections of the natural history of the HPV. In Section 5, we will perform a local sensitivity analysis of the basic reproductive number. This will be followed by a discussion of the results obtained and the conclusions, indicated in Sections 6 and 7, respectively.

## 2. Epithelial Cellular Dynamics

We assume that stratum spinosum and stratum granulosum cells have similar cell dynamics. Therefore, these cells belong to a stratum that we call stratum intermedium (see Figure 1). Consequently, the cell dynamic model of the homeostatic stratified epithelium is composed of the stratum basale, stratum intermedium, and stratum corneum. The dynamic is visualized in Figure 3.

The model is given by *B*_*H*_(*t*), *E*_*H*_(*t*), and *C*_*H*_(*t*), which denote stratum basale, stratum intermedium, and stratum corneum formed by uninfected cells, respectively. The cells of *B*_*H*_(*t*) proliferate (or lateral differentiation) at rate *r*_*B*_ considering a logistic growth, with a carrying capacity *K*_*B*_; these have suprabasal differentiation to *E*_*H*_(*t*) at rate *δ*_*B*_ and die at rate *μ*_*B*_. The dynamics of *E*_*H*_(*t*) is generated by suprabasal differentiation of *B*_*H*_(*t*) at a rate *δ*_*B*_. This population increases by cell proliferation, which is governed by logistic growth at a rate *r*_*E*_ and a carrying capacity at rate *K*_*E*_. These decrease by suprabasal differentiation at a rate *δ*_*E*_, and we assume that there is no natural death. Finally, the dynamics of *C*_*H*_(*t*) are generated by suprabasal differentiation of *E*_*H*_(*t*) at rate *δ*_*E*_ and shed from the epithelial tissue at a rate *μ*_*C*_. We arrive at the following mathematical model:

(1) $$\begin{array}{c} \frac{dB_{H}}{dt}=r_{B}B_{H}\left(1-\frac{B_{H}}{K_{B}}\right)-\delta_{B}B_{H}-\mu_{B}B_{H},\\ \frac{dE_{H}}{dt}=\delta_{B}B_{H}+r_{E}E_{H}\left(1-\frac{E_{H}}{K_{E}}\right)-\delta_{E}E_{H},\\ \frac{dC_{H}}{dt}=\delta_{E}E_{H}-\mu_{C}C_{H}. \end{array}$$

### 2.1. Positivity, Boundedness, Equilibria, and Their Local Stabilities

Let set *Ω*_*P*_ be *Ω*_*P*_ = {(*B*_*H*_, *E*_*H*_, *C*_*H*_) ∈ ℝ_+_^3^ : *B*_*H*_ ≥ 0, *E*_*H*_ ≥ 0, *C*_*H*_ ≥ 0} ⊂ ℝ^3^. We consider the positivity and boundedness of the solutions of system (1).

**Theorem 1 .**

Given the initial conditions *B*_*H*_(0) > 0, *E*_*H*_(0) > 0, *C*_*H*_(0) > 0, then all solutions of system (1) are positive.

**Proof**

At first, we will prove the positivity of *B*_*H*_(*t*). Let *B*_*H*_(0) be the solution that satisfies the initial condition *B*_*H*_(*t*) > 0. Assume that the solution is not always positive; i.e., there exists a *t*_0_′ ∈ ℝ_+_, such as *B*_*H*_(*t*_0_′) < 0. By Bolzano's theorem, there exists a *t*_1_ ∈ (0, *t*_0_′), such as *B*_*H*_(*t*_1_) = 0. Let *t*_0_ ∈ ℝ_+_ be the initial time, such as *B*_*H*_(*t*_0_) = 0, and then *dB*_*H*_(*t*)/*dt* = 0. Note that if some *t* ≥ 0, *B*_*H*_(*t*) = 0, then *dB*_*H*_(*t*)/*dt* = 0. Then, any solution with *B*_*H*_(0) = 0 will satisfy *B*_*H*_(*t*) = 0∀*t* > 0. By uniqueness of solutions, we have that if *B*_*H*_(0) > 0, then *B*_*H*_(*t*) will remain positive ∀*t* > 0. Therefore, *B*_*H*_(*t*_0_) = 0 leads to a contradiction. Hence, *B*_*H*_(*t*) is nonnegative for all *t* > 0. Now, we will prove the positivity of *E*_*H*_(*t*). *E*_*H*_(*t*) is not always positive; i.e., there exists *t*_0_′ ∈ ℝ_+_, such as *E*_*H*_(*t*_0_′) < 0. By Bolzano's theorem, there exists *t*_1_ ∈ (0, *t*_0_′), such as *E*_*H*_(*t*_1_) = 0. Let *t*_0_ = min{*t*_*i*_ | *E*_*H*_(*t*_*i*_) = 0}. By the second equation (1), if *E*_*H*_(*t*_0_) = 0, then *dE*_*H*_(*t*_0_)/*dt* = *δ*_*b*_*B*_*H*_ > 0 implies that *E*_*H*_ is increasing at *t* = *t*_0_. Therefore, *E*_*H*_(*t*) will be negative for values *t* < *t*_0_ near to *t*_0_, that is, a contradiction. Finally, we will prove the positivity of *C*_*H*_. From the third equation (1), we obtain the following inequality *dC*_*H*_(*t*)/*dt* ≥ −*μ*_*C*_*C*_*H*_(*t*). Integrating, we obtain the solution *C*_*H*_ ≥ *C*_*H*_(0)*e*^−*μt*^; therefore, *C*_*H*_ ≥ 0.

**Theorem 2 .**

Let (*B*_*H*_(*t*), *E*_*H*_(*t*), *C*_*H*_(*t*)) be the solution of model (1) with the initial conditions *B*_*H*_(0) > 0, *E*_*H*_(0) > 0, and *C*_*H*_(0) > 0. Then, *B*_*H*_(*t*), *E*_*H*_(*t*), and *C*_*H*_(*t*) are all bounded for all *t* ≥ 0 at which the solution exists.

**Proof**

Let (*B*_*H*_(*t*), *E*_*H*_(*t*), *C*_*H*_(*t*)) be any solution with nonnegative initial conditions. We define a function

(2) $$\begin{array}{c} B\left(t\right)=B_{H}\left(t\right)+E_{H}\left(t\right)+\left(\frac{n-1}{n}\right)C_{H}\left(t\right),n\gg 1. \end{array}$$

The time derivative along a solution of (2) is

(3) $$\begin{array}{c} \frac{dB\left(t\right)}{dt}=r_{B}B_{H}\left(1-\frac{B_{H}}{K_{B}}\right)-\mu_{B}B_{H}+r_{E}E_{H}\left(1-\frac{E_{H}}{K_{E}}\right)-\frac{\delta_{E}}{n}E_{H}-\mu_{C}\left(\frac{n-1}{n}\right)C_{H}=\frac{r_{B}K_{B}}{4}+\frac{r_{E}K_{E}}{4}-\mu_{B}B_{H}-\frac{\delta_{E}}{n}E_{H}-\mu_{C}\left(\frac{n-1}{n}\right)C_{H}-\frac{r_{B}}{K_{B}}{\left[B_{H}-\frac{K_{B}}{2}\right]}^{2}-\frac{r_{E}}{K_{E}}{\left[E_{H}-\frac{K_{E}}{2}\right]}^{2}\leq \frac{r_{B}K_{B}}{4}+\frac{r_{E}K_{E}}{4}-\mu_{B}B_{H}-\frac{\delta_{E}}{n}E_{H}-\mu_{C}\left(\frac{n-1}{n}\right)C_{H}. \end{array}$$

It follows that

(4) $$\begin{array}{c} \frac{dB\left(t\right)}{dt}+\eta B\left(t\right)\leq \frac{r_{B}K_{B}+r_{E}K_{E}}{4}, \end{array}$$

where *η* = min{*μ*_*B*_, *δ*_*E*_/*n*, *μ*_*C*_}. Thus, limsup_*t*⟶∞_*B*(*t*) ≤ (*r*_*B*_*K*_*B*_ + *r*_*E*_*K*_*E*_)/4*η*. Therefore, *B*_*H*_(*t*), *E*_*H*_(*t*), and *C*_*H*_(*t*) are all bounded for all *t* ≥ 0.

**Remark 1 .**

The total number of cervical epithelial cells is bounded by a weighted sum of the stratum basale and stratum intermedium carrying capacities, where the weights are the proliferation rates divided by four times of minimum of the death and differentiation rates. The above is biologically plausible that there is an upper bound in terms of the carrying capacities of the cells.

We can easily see that for all of the parameter values, the trivial equilibrium *E*_0_^1^ = (0, 0, 0) always exists. We get the “epithelial cell homeostasis” equilibrium *E*_1_^1^ = (*B*_*H*_^∗^, *E*_*H*_^∗^, *C*_*H*_^∗^), where

(5) $$\begin{array}{c} B_{H}^{*}=K_{B}\left(1-\frac{\delta_{B}+\mu_{B}}{r_{B}}\right), \end{array}$$

(6) $$\begin{array}{c} E_{H}^{*}=\frac{K_{E}}{2r_{E}}\left(r_{E}-\delta_{E}+\sqrt{{\left(\delta_{E}-r_{E}\right)}^{2}+4\frac{\delta_{B}r_{E}K_{B}}{K_{E}}\left(1-\frac{\delta_{B}+\mu_{B}}{r_{B}}\right)}\;\right), \end{array}$$

(7) $$\begin{array}{c} C_{H}^{*}=\frac{\delta_{E}}{\mu_{C}}E_{H}^{*}. \end{array}$$

The following inequality *r*_*B*_ > *δ*_*B*_ + *μ*_*B*_ is a biological condition for the maintenance of cell homeostasis of the epithelium.

The Jacobian matrix of (1) at *E*_0_^1^ is

(8) $$\begin{array}{c} J\left(E_{0}^{1}\right)=\left(\begin{array}{ccc} r_{B}-\delta_{B}-\mu_{B} & 0 & 0\\ \delta_{B} & r_{E}-\delta_{E} & 0\\ 0 & \delta_{E} & -\mu_{C} \end{array}\right). \end{array}$$

The eigenvalues of *J*(*E*_0_^1^) are *λ*_1_ = *r*_*B*_ − *δ*_*B*_ − *μ*_*B*_, *λ*_2_ = *r*_*E*_ − *δ*_*E*_, and *λ*_3_ = −*μ*_*C*_. By biological condition, *r*_*B*_ > *δ*_*B*_ + *μ*_*B*_, then *J*(*E*_0_^1^) has one positive eigenvalue. Thus, the trivial equilibrium is unstable.

The Jacobian matrix for the equations of (1) at *E*_1_^1^ is

(9) $$\begin{array}{c} J\left(E_{1}^{1}\right)=\left(\begin{array}{ccc} r_{B}\left(1-\frac{2B_{H}}{K_{B}}\right)-\delta_{B}-\mu_{B} & 0 & 0\\ \delta_{B} & r_{E}-\frac{2r_{E}E_{H}}{K_{E}}-\delta_{E} & 0\\ 0 & \delta_{E} & -\mu_{C} \end{array}\right). \end{array}$$

Using the following identities *r*_*B*_ − *r*_*B*_*B*_*H*_^∗^/*K*_*B*_ − (*δ*_*B*_ + *μ*_*B*_) = 0 and *r*_*E*_ − *r*_*E*_*E*_*H*_^∗^/*K*_*E*_ − *δ*_*E*_ = −*δ*_*B*_*B*_*H*_^∗^/*E*_*H*_^∗^, we have

(10) $$\begin{array}{c} J\left(E_{1}^{1}\right)=\left(\begin{array}{ccc} -\frac{B_{H}^{*}}{K_{B}} & 0 & 0\\ \delta_{B} & -\frac{\delta_{B}B_{H}^{*}}{E_{H}^{*}}-\frac{r_{E}E_{H}^{*}}{K_{E}} & 0\\ 0 & \delta_{E} & -\mu_{C} \end{array}\right). \end{array}$$

The characteristic polynomial of *J*(*E*_1_^1^) is

(11) $$\begin{array}{c} P\left(\lambda_{1}^{1}\right)=\left(\lambda_{1}^{1}-\left(-\frac{B_{H}^{*}}{K_{B}}\right)\right)\left(\lambda_{1}^{1}-\left(-\frac{\delta_{B}B_{H}^{*}}{E_{H}^{*}}-\frac{r_{E}E_{H}^{*}}{K_{E}}\right)\right)\left(\lambda_{1}^{1}-\left(-\mu_{C}\right)\right). \end{array}$$

The eigenvalues of *P*(*λ*_1_^1^) are *λ*_1,1_^1^ = −*B*_*H*_^∗^/*K*_*B*_, *λ*_1,2_^1^ = −*δ*_*B*_*B*_*H*_^∗^/*E*_*H*_^∗^ − *r*_*E*_*E*_*H*_^∗^/*K*_*E*_, and *λ*_1,3_^1^ = −*μ*_*C*_. Clearly, all of the eigenvalues are negative. Consequently, the epithelial cell homeostasis equilibrium *E*_1_^1^ is locally asymptotically stable.

We then arrive at the following theorem.

**Theorem 3 .**

Assume that the biological condition *r*_*B*_ > *δ*_*B*_ + *μ*_*B*_ is satisfied. The trivial equilibrium *E*_0_^1^ = (0, 0, 0) always exists and is unstable. The epithelial cell homeostasis equilibrium *E*_1_^1^ = (*B*_*H*_^∗^, *E*_*H*_^∗^, *C*_*H*_^∗^) always exists and is absolutely stable.

### 2.2. Global Stability of the Epithelial Cell Homeostasis Equilibrium

We use the method of Lyapunov functions and a theorem on limiting systems to analyze the global stability of the epithelial cell homeostasis equilibrium of the system (1).

Consider the *B*_*H*_ − *E*_*H*_ subsystem of model (1), which is independent of the *C*_*H*_ variables. We construct the following Volterra-type Lyapunov function [26] for the *B*_*H*_ − *E*_*H*_ subsystem

(12) $$\begin{array}{c} U\left(t\right)=2\int_{B_{H}^{*}}^{B_{H}}\left(1-\frac{B_{H}^{*}}{\eta }\right)d\eta +\frac{r_{B}}{\delta_{B}K_{B}}\int_{E_{H}^{*}}^{E_{H}}\left(1-\frac{E_{H}^{*}}{\eta }\right)d\eta . \end{array}$$

The function *U*(*t*) is defined, continuous, and positive definite for all *B*_*H*_, *E*_*H*_ > 0. Also, the global minimum *U*(*B*_*H*_, *E*_*H*_) = 0 occurs at (*B*_*H*_^∗^, *E*_*H*_^∗^), and therefore, *U* is a Lyapunov function. First, we calculate the time derivative of *U*(*t*) computed along solutions of the first two equations of the system (1), given by the expression

(13) $$\begin{array}{c} \frac{dU\left(t\right)}{dt}=2\left(1-\frac{B_{H}^{*}}{B_{H}}\right)\frac{dB_{H}}{dt}+\frac{r_{B}}{\delta_{B}K_{B}}\left(1-\frac{E_{H}^{*}}{E_{H}}\right)\frac{dE_{H}}{dt}. \end{array}$$

Note that

(14) $$\begin{array}{c} 1=\frac{B_{H}^{*}}{K_{B}}+\frac{\delta_{B}+\mu_{B}}{r_{B}}, \end{array}$$

(15) $$\begin{array}{c} 1=\frac{\delta_{E}}{r_{E}}-\frac{\delta_{B}}{r_{E}}\frac{B_{H}^{*}}{E_{H}^{*}}+\frac{E_{H}^{*}}{K_{E}}. \end{array}$$

Using (14) and (15), we have

(16) $$\begin{array}{c} \frac{dU\left(t\right)}{dt}=\left(1-\frac{B_{H}^{*}}{B_{H}}\right)\left[r_{B}\frac{B_{H}^{*}}{K_{B}}B_{H}\left(1-\frac{B_{H}}{B_{H}^{*}}\right)\right]+\left(1-\frac{B_{H}^{*}}{B_{H}}\right)\left[r_{B}\frac{B_{H}^{*}}{K_{B}}B_{H}\left(1-\frac{B_{H}}{B_{H}^{*}}\right)\right]+\frac{r_{B}}{\delta_{B}K_{B}}\left(1-\frac{E_{E}^{*}}{E_{H}}\right)\left[\delta_{B}B_{H}^{*}\left(\frac{B_{H}}{B_{H}^{*}}-\frac{E_{H}}{E_{H}^{*}}\right)+r_{E}E_{H}\frac{E_{H}^{*}}{K_{E}}\left(1-\frac{E_{H}}{E_{H}^{*}}\right)\right]=r_{B}B_{H}\frac{B_{H}^{*}}{K_{B}}\left(2-\frac{B_{H}}{B_{H}^{*}}-\frac{B_{H}^{*}}{B_{H}}\right)+\frac{r_{B}}{\delta_{B}K_{B}}r_{E}E_{H}\frac{E_{H}^{*}}{K_{E}}\left(2-\frac{E_{H}}{E_{H}^{*}}-\frac{E_{H}^{*}}{E_{H}}\right)+r_{B}\frac{B_{H}^{*}}{K_{B}}\left(3-\frac{B_{H}^{*}}{B_{H}}-\frac{E_{H}}{E_{H}^{*}}-\frac{B_{H}E_{E}^{*}}{B_{H}^{*}E_{H}}\right)<-\frac{r_{B}}{K_{B}}{\left(B_{H}-B_{H}^{*}\right)}^{2}-\frac{r_{B}}{\delta_{B}K_{B}}\frac{r_{E}}{K_{E}}{\left(E_{H}-E_{H}^{*}\right)}^{2}. \end{array}$$

Because *dU*(*t*)/*dt* ≤ 0, the Lyapunov stability theorem [27] implies that the (*B*_*H*_^∗^, *E*_*H*_^∗^) equilibrium is globally asymptotically stable in ℝ_+_^2^ and lim_*t*⟶∞_*E*_*H*_(*t*) = *E*_*H*_^∗^.

From the third equation in (1), we can formally solve to obtain

(17) $$\begin{array}{c} C_{H}\left(t\right)=\left[C_{H}\left(0\right)+\int_{t_{0}}^{t}\delta_{E}E_{H}\left(\tau \right)e^{\mu_{C}\left(\tau -t_{0}\right)}d\tau \right]/e^{\mu_{C}\left(t-t_{0}\right)}. \end{array}$$

By L'Hospital's rule, we obtain lim_*t*⟶∞_*C*_*H*_(*t*) = *δ*_*E*_*E*_*H*_/*μ*_*C*_ = *δ*_*E*_*E*_*H*_^∗^/*μ*_*C*_ = *C*_*H*_^∗^. An application of Lemma 1 [28] shows that the epithelial cell homeostasis equilibrium *E*_1_^1^ = (*B*_*H*_^∗^, *E*_*H*_^∗^, *C*_*H*_^∗^) of model (1) is globally asymptotically stable in the interior of *Ω*_*P*_. We then have the following theorem.

**Theorem 4 .**

If *r*_*B*_ > *δ*_*B*_ + *μ*_*B*_, then the epithelial cell homeostasis equilibrium *E*_1_^1^ = (*B*_*H*_^∗^, *E*_*H*_^∗^, *C*_*H*_^∗^) of system (1) is globally asymptotically stable in the interior of *Ω*_*P*_.

## 3. Epithelial Viral Dynamics of HPV

The viral dynamics model includes that of uninfected cells, infected cells, and viral load. The viral dynamics are given by *B*_*I*_(*t*), *E*_*I*_(*t*), *C*_*I*_(*t*), and *V*(*t*), which denote the cells of the stratum basale, stratum intermedium, stratum corneum infected, and the viral load, respectively. *B*_*H*_(*t*), *E*_*H*_(*t*), and *C*_*H*_(*t*) are denoted in the same way as in the previous section.

Figure 4 shows that the dynamics of *B*_*I*_(*t*) results from contact between uninfected basal cells and HPV particle at rate *β*. This population increases by cell proliferation (or lateral differentiation), governed by full logistic growth at a rate *r*_*B*_^∗^, and a carrying capacity at rate *K*_*B*_. These decrease by suprabasal differentiation at rate *δ*_*B*_^∗^ and death cellular at rate *μ*_*B*_^∗^. The dynamics of *E*_*I*_(*t*) are generated by suprabasal differentiation of *B*_*I*_(*t*) at a rate *δ*_*B*_^∗^. This population increases by cell proliferation, governed by full logistic growth at a rate *r*_*E*_^∗^, and a carrying capacity at rate *K*_*E*_. These decrease by suprabasal differentiation at a rate *δ*_*E*_^∗^, and we assume that there is no natural death. The dynamics of *C*_*I*_(*t*) are generated by suprabasal differentiation of *E*_*I*_(*t*) at rate *δ*_*E*_^∗^. There is no proliferation of *C*_*I*_(*t*). This population decreases by desquamation at rate *μ*_*C*_^∗^. Finally, *V*(*t*) increases by rupture of cell membrane of *C*_*I*_(*t*) at rate *σ*, and they decline at rate *γ*. This is summarized in the following nonlinear ODE system:

(18) $$\begin{array}{c} \frac{dB_{H}}{dt}=r_{B}B_{H}\left(1-\frac{B_{H}+B_{I}}{K_{B}}\right)-\delta_{B}B_{H}-\mu_{B}B_{H}-\beta B_{H}V,\\ \frac{dB_{I}}{dt}=\beta B_{H}V+r_{B}^{*}B_{I}\left(1-\frac{B_{H}+B_{I}}{K_{B}}\right)-\delta_{B}^{*}B_{I}-\mu_{B}^{*}B_{I},\\ \frac{dE_{H}}{dt}=\delta_{B}B_{H}+r_{E}E_{H}\left(1-\frac{E_{H}+E_{I}}{K_{E}}\right)-\delta_{E}E_{H},\\ \frac{dE_{I}}{dt}=\delta_{B}^{*}B_{I}+r_{E}^{*}E_{I}\left(1-\frac{E_{H}+E_{I}}{K_{E}}\right)-\delta_{E}^{*}E_{I},\\ \frac{dC_{H}}{dt}=\delta_{E}E_{H}-\mu_{C}C_{H},\\ \frac{dC_{I}}{dt}=\delta_{E}^{*}E_{I}-\mu_{C}^{*}C_{I},\\ \frac{dV\;}{dt}=\sigma C_{I}-\gamma V. \end{array}$$

### 3.1. Positivity, Boundedness, Equilibria, Basic Reproductive Number, and Local Stability

Let set *Ω*_*G*_ be *Ω*_*G*_ = {(*B*_*H*_, *B*_*I*_, *E*_*H*_, *E*_*I*_, *C*_*H*_, *C*_*I*_, *V*) ∈ ℝ_+_^7^ : *B*_*H*_ ≥ 0, *B*_*I*_ ≥ 0, *E*_*H*_ ≥ 0, *E*_*I*_ ≥ 0, *C*_*H*_ ≥ 0, *C*_*I*_ ≥ 0, *V* ≥ 0} ⊂ ℝ^7^. We consider the positivity and boundedness of the solutions of system (18).

**Theorem 5 .**

Given the initial conditions *B*_*H*_(0) > 0, *B*_*I*_(0) ≥ 0, *E*_*H*_(0) > 0, *E*_*I*_(0) ≥ 0, *C*_*H*_(0) > 0, *C*_*H*_(0) ≥ 0 and *V*(0) > 0, then all solutions of system (18) are positive.

The proof of Theorem 1 is very similar to the proof of Theorem 6. For this reason, we omit the proof.

**Theorem 6 .**

Let (*B*_*H*_(*t*), *B*_*I*_(*t*), *E*_*H*_(*t*), *E*_*I*_(*t*), *C*_*H*_(*t*), *C*_*I*_(*t*), *V*(*t*)) be the solution of model (18) with the initial conditions *B*_*H*_(0) > 0, *B*_*I*_(0) ≥ 0, *E*_*H*_(0) > 0, *E*_*I*_(0) ≥ 0, *C*_*H*_(0) > 0, *C*_*H*_(0) ≥ 0 and *V*(0) > 0. Then, *B*_*H*_(*t*), *B*_*I*_(*t*), *E*_*H*_(*t*), *E*_*I*_(*t*), *C*_*H*_(*t*), *C*_*I*_(*t*), and *V*(*t*) are all bounded for all *t* ≥ 0 at which the solution exists.

**Proof**

Let (*B*_*H*_(*t*), *B*_*I*_(*t*), *E*_*H*_(*t*), *E*_*I*_(*t*), *C*_*H*_(*t*), *C*_*I*_(*t*), *V*(*t*)) be any solution with nonnegative initial conditions. We define a function

(19) $$\begin{array}{c} B\left(t\right)=B_{H}\left(t\right)+B_{I}\left(t\right)+E_{H}\left(t\right)+E_{I}\left(t\right)+\left(\frac{n}{n+1}\right)C_{H}\left(t\right)+\left(\frac{n}{n+1}\right)C_{I}\left(t\right)+\left(\frac{\mu_{C}^{*}\left(n-1\right)}{\sigma \left(n+1\right)}\right)V\left(t\right),n\gg 1. \end{array}$$

The time derivative along a solution of (19) is

(20) $$\begin{array}{c} \frac{dB\left(t\right)}{dt}=r_{B}B_{H}\left(1-\frac{B_{H}}{K_{B}}\right)+r_{B}^{*}B_{I}\left(1-\frac{B_{I}}{K_{B}}\right)+r_{E}E_{H}\left(1-\frac{E_{H}}{K_{E}}\right)+r_{E}^{*}E_{I}\left(1-\frac{E_{I}}{K_{E}}\right)-\frac{r_{B}+r_{B}^{*}}{K_{B}}B_{H}B_{I}-\frac{r_{E}+r_{E}^{*}}{K_{E}}E_{H}E_{I}-\mu_{B}B_{H}-\mu_{B}^{*}B_{I}-\frac{\delta_{E}}{n+1}E_{H}-\frac{\delta_{E}^{*}}{n+1}E_{I}-\mu_{C}\left(\frac{n}{n+1}\right)C_{H}-\frac{\mu_{C}^{*}}{n}\left(\frac{n}{n+1}\right)C_{I}-\gamma \left(\frac{\mu_{C}^{*}\left(n-1\right)}{\sigma \left(n+1\right)}\right)V\left(t\right)=\frac{\left(r_{B}+r_{B}^{*}\right)K_{B}}{4}+\frac{\left(r_{E}+r_{E}^{*}\right)K_{E}}{4}-\frac{r_{B}}{K_{B}}{\left[B_{H}-\frac{K_{B}}{2}\right]}^{2}-\frac{r_{B}^{*}}{K_{B}}{\left[B_{I}-\frac{K_{B}}{2}\right]}^{2}-\frac{r_{E}}{K_{E}}{\left[E_{H}-\frac{K_{E}}{2}\right]}^{2}-\frac{r_{E}^{*}}{K_{E}}{\left[E_{I}-\frac{K_{E}}{2}\right]}^{2}-\frac{r_{B}+r_{B}^{*}}{K_{B}}B_{H}B_{I}-\frac{r_{E}+r_{E}^{*}}{K_{E}}E_{H}E_{I}-\mu_{B}B_{H}-\mu_{B}^{*}B_{I}-\frac{\delta_{E}}{n+1}E_{H}-\frac{\delta_{E}^{*}}{n+1}E_{I}-\mu_{C}\left(\frac{n}{n+1}\right)C_{H}-\frac{\mu_{C}^{*}}{n}\left(\frac{n}{n+1}\right)C_{I}-\gamma \left(\frac{\mu_{C}^{*}\left(n-1\right)}{\sigma \left(n+1\right)}\right)V\left(t\right)\leq \frac{\left(r_{B}+r_{B}^{*}\right)K_{B}+\left(r_{E}+r_{E}^{*}\right)K_{E}}{4}-\mu_{B}B_{H}-\mu_{B}^{*}B_{I}-\frac{\delta_{E}}{n+1}E_{H}-\frac{\delta_{E}^{*}}{n+1}E_{I}-\mu_{C}\left(\frac{n}{n+1}\right)C_{H}-\frac{\mu_{C}^{*}}{n}\left(\frac{n}{n+1}\right)C_{I}-\gamma \left(\frac{\mu_{C}^{*}\left(n-1\right)}{\sigma \left(n+1\right)}\right)V\left(t\right). \end{array}$$

It follows that

(21) $$\begin{array}{c} \frac{dB\left(t\right)}{dt}+\eta B\left(t\right)\leq \frac{\left(r_{B}+r_{B}^{*}\right)K_{B}+\left(r_{E}+r_{E}^{*}\right)K_{E}}{4}, \end{array}$$

where *η* = min{*μ*_*B*_, *μ*_*B*_^∗^, *δ*_*E*_/(*n* + 1), *δ*_*E*_^∗^/(*n* + 1), *μ*_*C*_, *μ*_*C*_^∗^/*n*, *γ*}. Thus, limsup_*t*⟶∞_*B*(*t*) ≤ ((*r*_*B*_ + *r*_*B*_^∗^)*K*_*B*_ + (*r*_*E*_ + *r*_*E*_^∗^)*K*_*E*_)/4*η*. Therefore, *B*_*H*_(*t*), *B*_*I*_(*t*), *E*_*H*_(*t*), *E*_*I*_(*t*), *C*_*H*_(*t*), *C*_*I*_(*t*), and *V*(*t*) are all bounded for all *t* ≥ 0.

**Remark 2 .**

The total number of cervical epithelial cells, both uninfected and infected, and viral load is bounded by a weighted sum of the stratum basale and stratum intermedium carrying capacities, where the weights are the proliferation rates of healthy and infected cells divided by four times of minimum of the death, differentiation, and viral clearance rates.

The model (18) always have a trivial equilibrium *E*_0_^2^ = (0, 0, 0, 0, 0, 0, 0), and a “epithelial cell homeostasis” equilibrium *E*_1_^2^ = (*B*_*H*_^∗^, 0, *E*_*H*_^∗^, 0, *C*_*H*_^∗^, 0, 0) with the same coordinates *B*_*H*_^∗^, *E*_*H*_^∗^, and *C*_*H*_^∗^ given in (5), (6) and (7), respectively. We recall the “epithelial cell homeostasis” equilibrium as the infection-free equilibrium.

The Jacobian matrix of system (18) is

(22) $$\begin{array}{c} J=\left(\begin{array}{ccccccc} J_{11} & -\frac{r_{B}B_{H}}{K_{B}} & 0 & 0 & 0 & 0 & -\beta B_{H}\\ \beta V-\frac{r_{B}^{*}B_{I}}{K_{B}} & J_{22} & 0 & 0 & 0 & 0 & \beta B_{H}\\ \delta_{B} & 0 & J_{33} & -\frac{r_{E}E_{H}}{K_{E}} & 0 & 0 & 0\\ 0 & \delta_{B}^{*} & -\frac{r_{E}^{*}E_{I}}{K_{E}} & J_{44} & 0 & 0 & 0\\ 0 & 0 & \delta_{E} & 0 & -\mu_{C} & 0 & 0\\ 0 & 0 & 0 & \delta_{E}^{*} & 0 & -\mu_{C}^{*} & 0\\ 0 & 0 & 0 & 0 & 0 & \sigma & -\gamma \end{array}\right), \end{array}$$

where

(23) $$\begin{array}{c} J_{11}=r_{B}-\frac{2r_{B}}{K_{B}}B_{H}-\frac{r_{B}}{K_{B}}B_{I}-\delta_{B}-\mu_{B}-\beta V,\\ J_{22}=r_{B}^{*}-\frac{r_{B}^{*}}{K_{B}}B_{H}-\frac{2r_{B}^{*}}{K_{B}}B_{I}-\delta_{B}^{*}-\mu_{B}^{*},\\ J_{33}=r_{E}-\frac{2r_{E}}{K_{E}}E_{H}-\frac{r_{E}}{K_{E}}E_{I}-\delta_{E},\\ J_{44}=r_{E}^{*}-\frac{r_{E}^{*}}{K_{E}}E_{H}-\frac{2r_{E}^{*}}{K_{E}}E_{I}-\delta_{E}^{*}. \end{array}$$

#### 3.1.1. Basic Reproductive Number *R*_0_

To compute the basic reproductive number *R*_0_, we use the next-generation operator introduced by van den Driessche and Watmough [29]. The Jacobian matrix *J* of this subsystem at the infection-free equilibrium is decomposed as *J* = *F* − *V*, where *F* is the viral transmission part and *V* describe the transition terms associated with the model (18). These quantities are given, respectively, by

(24) $$\begin{array}{c} F≔\left(\begin{array}{cccc} r_{B}^{*}\left(1-\frac{B_{H}^{*}}{K_{B}}\right) & 0 & 0 & \beta B_{H}^{*}\\ 0 & 0 & 0 & 0\\ 0 & 0 & 0 & 0\\ 0 & 0 & 0 & 0 \end{array}\right),\\ V≔\left(\begin{array}{cccc} \delta_{B}^{*}+\mu_{B}^{*} & 0 & 0 & 0\\ -\delta_{B}^{*} & \delta_{E}^{*}-r_{E}^{*}\left(1-\frac{E_{H}^{*}}{K_{E}}\right) & 0 & 0\\ 0 & -\delta_{E}^{*} & \mu_{C}^{*} & 0\\ 0 & 0 & -\sigma & \gamma \end{array}\right). \end{array}$$

It follows that the basic reproductive number *R*_0_ = *ρ*(*FV*^−1^), where *ρ* is the spectral radius, is given by

(25) $$\begin{array}{c} R_{0}=\frac{1}{\delta_{B}^{*}+\mu_{B}^{*}}\left[\frac{\beta \sigma \delta_{B}^{*}\delta_{E}^{*}B_{H}^{*}}{\gamma \mu_{C}^{*}\left(\delta_{E}^{*}-r_{E}^{*}\left(1-E_{H}^{*}/K_{E}\right)\right)}+r_{B}^{*}\left(1-\frac{B_{H}^{*}}{K_{B}}\right)\right]. \end{array}$$

The parameter *R*_0_ has an interesting biological meaning: it is the sum of average numbers of secondary infected cells produced by a single infected cell in a population of epithelial basal cells, by direct basal cell-to-HPV contact and infected basal cell division, respectively.

**Remark 3 .**

If *r*_*E*_^∗^(1 − *E*_*H*_^∗^/*K*_*E*_) is taken as a new infection, we can get another basic reproductive number as follows:

(26) $$\begin{array}{c} {\bar{R}}_{0}=\frac{1}{2}\left(a+b+c\right)+\frac{1}{2}\sqrt{a^{2}+{\left(b-c\right)}^{2}+2a\left(b+c\right)}, \end{array}$$

where

(27) $$\begin{array}{c} a=\frac{\beta \sigma \delta_{B}^{*}B_{H}^{*}}{\gamma \mu_{C}^{*}\left(\delta_{B}^{*}+\mu_{B}^{*}\right)},\\ b=\frac{r_{B}^{*}}{\delta_{B}^{*}+\mu_{B}^{*}}\left(1-\frac{B_{H}^{*}}{K_{B}}\right),\\ c=\frac{r_{E}^{*}}{\delta_{E}^{*}}\left(1-\frac{E_{H}^{*}}{K_{E}}\right). \end{array}$$

When *r*_*E*_^∗^ = 0, it is easy to check that *R*_0_ is equivalent to ${\bar{R}}_{0}$.

#### 3.1.2. Local Stability of *E*_0_^2^

The Jacobian matrix (22) evaluated at the equilibrium point *E*_0_^2^ becomes

(28) $$\begin{array}{c} J\left(E_{0}^{2}\right)=\left(\begin{array}{ccccccc} r_{B}-\delta_{B}-\mu_{B} & 0 & 0 & 0 & 0 & 0 & 0\\ 0 & r_{B}^{*}-\delta_{B}^{*}-\mu_{B}^{*} & 0 & 0 & 0 & 0 & 0\\ \delta_{B} & 0 & r_{E}-\delta_{E} & 0 & 0 & 0 & 0\\ 0 & \delta_{B}^{*} & 0 & r_{E}^{*}-\delta_{E}^{*} & 0 & 0 & 0\\ 0 & 0 & \delta_{B} & 0 & -\mu_{C} & 0 & 0\\ 0 & 0 & 0 & \delta_{B}^{*} & 0 & -\mu_{C}^{*} & 0\\ 0 & 0 & 0 & 0 & 0 & \sigma & -\gamma \end{array}\right). \end{array}$$

By the biological condition, one of its eigenvalues is positive:

(29) $$\begin{array}{c} \lambda_{0,1}^{2}=r_{B}-\delta_{B}-\mu_{B}>0, \end{array}$$

while the other six are

(30) $$\begin{array}{c} \begin{array}{c} \lambda_{0,2}^{2}=r_{E}-\delta_{E},\\ \lambda_{0,3}^{2}=r_{B}^{*}-\delta_{B}^{*}-\mu_{B}^{*},\\ \lambda_{0,4}^{2}=r_{E}^{*}-\delta_{E}^{*},\\ \lambda_{0,5}^{2}=-\mu_{C},\\ \lambda_{0,6}^{2}=-\mu_{C}^{*},\\ \lambda_{0,7}^{2}=-\gamma . \end{array} \end{array}$$

Thus, *E*_0_^2^ is unstable. This result can be summarized as follows.

**Theorem 7 .**

Assume that the biological condition *r*_*B*_ > *δ*_*B*_ + *μ*_*B*_ is satisfied. The trivial equilibrium *E*_0_^2^ = (0, 0, 0, 0, 0, 0, 0) always exists and is unstable.

#### 3.1.3. Local Stability of *E*_1_^2^

The Jacobian matrix of system (18), evaluated in the infection-free equilibrium point *E*_1_^2^, takes the form

(31) $$\begin{array}{c} J\left(E_{1}^{2}\right)=\left(\begin{array}{ccccccc} J_{11} & -\frac{r_{B}}{K_{B}}B_{H}^{*} & 0 & 0 & 0 & 0 & -\beta B_{H}^{*}\\ 0 & J_{22} & 0 & 0 & 0 & 0 & \beta B_{H}^{*}\\ \delta_{B} & 0 & J_{33} & -\frac{r_{E}}{K_{E}}E_{H}^{*} & 0 & 0 & 0\\ 0 & \delta_{B}^{*} & 0 & J_{44} & 0 & 0 & 0\\ 0 & 0 & \delta_{E} & 0 & -\mu_{C} & 0 & 0\\ 0 & 0 & 0 & \delta_{E}^{*} & 0 & -\mu_{C}^{*} & 0\\ 0 & 0 & 0 & 0 & 0 & \sigma & -\gamma \end{array}\right) \end{array}$$

where

(32) $$\begin{array}{c} J_{11}=\left(r_{B}-\delta_{B}-\mu_{B}\right)-\frac{2r_{B}}{K_{B}}B_{H}^{*},\\ J_{22}=\left(r_{B}^{*}-\delta_{B}^{*}-\mu_{B}^{*}\right)-\frac{r_{B}^{*}}{K_{B}}B_{H}^{*},\\ J_{33}=\left(r_{E}-\delta_{E}\right)-\frac{2r_{E}}{K_{E}}E_{H}^{*},\\ J_{44}=\left(r_{E}^{*}-\delta_{E}^{*}\right)-\frac{r_{E}^{*}}{K_{E}}E_{H}^{*}. \end{array}$$

Using the following identities *r*_*B*_ − *r*_*B*_*B*_*H*_^∗^/*K*_*B*_ − (*δ*_*B*_ + *μ*_*B*_) = 0 and *r*_*E*_ − *r*_*E*_*E*_*H*_^∗^/*K*_*E*_ − *δ*_*E*_ = −*δ*_*B*_*B*_*H*_^∗^/*E*_*H*_^∗^, we have

(33) $$\begin{array}{c} J_{11}=-\left(r_{B}-\delta_{B}-\mu_{B}\right), \end{array}$$

(34) $$\begin{array}{c} J_{22}=\left(r_{B}^{*}-\delta_{B}^{*}-\mu_{B}^{*}\right)-\frac{r_{B}^{*}}{r_{B}}\left(r_{B}-\delta_{B}-\mu_{B}\right), \end{array}$$

(35) $$\begin{array}{c} J_{33}=-\frac{\delta_{B}B_{H}^{*}}{E_{H}^{*}}-\frac{r_{E}}{K_{E}}E_{H}^{*}, \end{array}$$

(36) $$\begin{array}{c} J_{44}=\left(r_{E}^{*}-\delta_{E}^{*}\right)-\frac{r_{E}^{*}}{r_{E}}\left(r_{E}-\delta_{E}\right)-\frac{r_{E}^{*}}{r_{E}}\frac{\delta_{B}B_{H}^{*}}{E_{H}^{*}}. \end{array}$$

By biological condition, *r*_*B*_ > *δ*_*B*_ + *μ*_*B*_, then *J*_11_ < 0 and *J*_33_ < 0. Furthermore, if

(37) $$\begin{array}{c} \frac{r_{B}^{*}}{\delta_{B}^{*}+\mu_{B}^{*}}\leq \frac{r_{B}}{\delta_{B}+\mu_{B}}, \end{array}$$

(38) $$\begin{array}{c} \frac{r_{E}^{*}}{\delta_{E}^{*}}<\frac{r_{E}}{\delta_{E}}, \end{array}$$

then *J*_22_ ≤ 0 and *J*_44_ < 0, respectively.

On the other hand, the characteristic polynomial of (31) is given by

(39) $$\begin{array}{c} P\left(\lambda_{1}^{2}\right)=\left(\mu_{C}+\lambda_{1}^{2}\right)\left(J_{33}-\lambda_{1}^{2}\right)\left(J_{11}-\lambda_{1}^{2}\right)\left({\left(\lambda_{1}^{2}\right)}^{4}+a_{1}{\left(\lambda_{1}^{2}\right)}^{3}+a_{2}{\left(\lambda_{1}^{2}\right)}^{2}+a_{3}\left(\lambda_{1}^{2}\right)+a_{4}\right), \end{array}$$

where

(40) $$\begin{array}{c} a_{1}\equiv \mu_{C}^{*}+\gamma -\left(J_{22}+J_{44}\right), \end{array}$$

(41) $$\begin{array}{c} a_{2}\equiv J_{22}J_{44}+\gamma \mu_{C}^{*}-\left(\gamma +\mu_{C}^{*}\right)\left(J_{22}+J_{44}\right), \end{array}$$

(42) $$\begin{array}{c} a_{3}\equiv \left(\mu_{C}^{*}+\gamma \right)J_{22}J_{44}-\gamma \mu_{C}^{*}\left(J_{22}+J_{44}\right), \end{array}$$

(43) $$\begin{array}{c} a_{4}\equiv \gamma J_{22}J_{44}\mu_{C}^{*}-\sigma \beta B_{H}^{*}\delta_{B}^{*}\delta_{E}^{*}=\gamma \mu_{C}^{*}\left(\delta_{B}^{*}+\mu_{B}^{*}\right)J_{44}\left(R_{0}-1\right). \end{array}$$

Note that in (43), *a*_4_ = 0 when *J*_44_ ≠ 0 and *R*_0_ = 1; consequently, one of the roots of (39) is zero. Therefore, in this case the equilibrium point *E*_1_^2^ has a zero eigenvalue, that is, it is no-hyperbolic.

Three eigenvalues of characteristic polynomial (39) are *λ*_1,1_^2^ = −*μ*_*C*_ < 0, *λ*_1,2_^2^ = *J*_33_ < 0 and *λ*_1,3_^2^ = *J*_11_ < 0. To determine the sign of the other four, which are the roots of the quadratic equation in (39), we will use the Ruth-Hurwitz criterion. According to this, such polynomial has roots with negative real part if and only if all its coefficients *a*_1_, *a*_2_, *a*_3_, and *a*_4_ are positive and the relations

(44) $$\begin{array}{c} a_{1}a_{2}>a_{3}, \end{array}$$

(45) $$\begin{array}{c} a_{1}a_{2}a_{3}>a_{4}a_{1}^{2}+a_{3}^{2}, \end{array}$$

hold. In order to show these relations, we will adopt the following notation:

(46) $$\begin{array}{c} A\equiv \gamma +\mu_{C}^{*}, \end{array}$$

(47) $$\begin{array}{c} B\equiv -\left(J_{22}+J_{44}\right), \end{array}$$

(48) $$\begin{array}{c} C\equiv \gamma \mu_{C}^{*}, \end{array}$$

(49) $$\begin{array}{c} D\equiv J_{22}J_{44}, \end{array}$$

(50) $$\begin{array}{c} E\equiv \sigma \beta B_{H}^{*}\delta_{B}^{*}\delta_{E}^{*}. \end{array}$$

Note that quantities *A* > 0 and *C* > 0, since *γ* and *μ*_*C*_^∗^ are positive parameters, and *E* is also positive. By the inequalities (37) and (38), we have that *B* is positive and *D* is nonnegative. Thus, in terms of this new notation, the quantities (40)–(43) can be rewritten as

(51) $$\begin{array}{c} a_{1}=A+B,\\ a_{2}=C+D+AB,\\ a_{3}=AD+BC,\\ a_{4}=CD-E. \end{array}$$

We note that the coefficients *a*_1_, *a*_2_, and *a*_3_ are positive, while if *J*_44_ < 0 (or equivalently *r*_*E*_^∗^/*δ*_*E*_^∗^ < *r*_*E*_/*δ*_*E*_) and *R*_0_ < 1 also, *a*_4_ is positive.

Thus, the condition of Ruth-Hurwitz (44) can be written as

(52) $$\begin{array}{c} \left(A+B\right)\left(C+D+AB\right)>AD+BC. \end{array}$$

First of all notice that from (46), *A*^2^ = *γ*^2^ + 2*C* + (*μ*_*C*_^∗^)^2^ > 2*C* > *C* and *B*^2^ = *J*_22_^2^ + 2*D* + *J*_44_^2^ > 2*D* > *D*. In this way, taking into account that *A* > 0 and *B* > 0, from the above inequalities, we get *BA*^2^ > *BC* and *AB*^2^ > *AD*. This result allows us to establish that

(53) $$\begin{array}{c} AB^{2}+BA^{2}>AD+BC. \end{array}$$

Expanding the left hand side of (52), this can be rewritten as

(54) $$\begin{array}{c} AB^{2}+A^{2}B+AD+BD+AC+BC>2AD+2BC+BD+AC. \end{array}$$

In (54), *AC* > 0 since *A* and *C* are positive definite, *BC* > 0 since that *B* > 0, and *AD* ≥ 0 and *BD* ≥ 0 since that *D* ≥ 0. We would have on the right hand side of (54) that 2*AD* + 2*BC* + *BD* + *AC* > 2*AD* + 2*BC* > *AD* + *BC*. Therefore, (52) is satisfied; that is, the inequality (44) holds.

On the other hand, the last condition of Ruth-Hurwitz (45) can be written as

(55) $$\begin{array}{c} \left(A+B\right)\left(C+D+AB\right)\left(AD+BC\right)>\left(CD-E\right){\left(A+B\right)}^{2}+{\left(AD+BC\right)}^{2}. \end{array}$$

The left side of (55) can be rewritten as

(56) $$\begin{array}{c} \left(A+B\right)\left(C+D+AB\right)\left(AD+BC\right)=\left[AB^{2}+A^{2}B+\left(C+D\right)\left(A+B\right)\right]\left(AD+BC\right). \end{array}$$

Note that the first factor on the right hand side of (56), taking (53) into account, takes the form

(57) $$\begin{array}{c} AB^{2}+A^{2}B+\left(C+D\right)\left(A+B\right)>\left(AD+BC\right)+\left(C+D\right)\left(A+B\right). \end{array}$$

Thus, the right hand side of (56) becomes

(58) $$\begin{array}{c} \left[AB^{2}+A^{2}B+\left(C+D\right)\left(A+B\right)\right]\left(AD+BC\right)>{\left(AD+BC\right)}^{2}+\left(C+D\right)\left(A+B\right)\left(AD+BC\right). \end{array}$$

Besides, the second term on the right hand side of (58) can be written as

(59) $$\begin{array}{c} \left(C+D\right)\left(A+B\right)\left(AD+BC\right)=A^{2}CD+A^{2}D^{2}+ABC^{2}+2ABCD+ABD^{2}+B^{2}C^{2}+B^{2}CD={\left(A+B\right)}^{2}CD+\left(BC^{2}+AD^{2}\right)\left(A+B\right)>{\left(A+B\right)}^{2}CD>{\left(A+B\right)}^{2}\left(CD-E\right), \end{array}$$

since *E* > 0, that is,

(60) $$\begin{array}{c} \left(C+D\right)\left(A+B\right)\left(AD+BC\right)>{\left(A+B\right)}^{2}\left(CD-E\right). \end{array}$$

Thus, from equations (56), (58), and (60), we have

(61) $$\begin{array}{c} \left(A+B\right)\left(C+D+AB\right)\left(AD+BC\right)=\left[AB^{2}+A^{2}B+\left(C+D\right)\left(A+B\right)\right]\left(AD+BC\right)>{\left(AD+BC\right)}^{2}+\left(C+D\right)\left(A+B\right)\left(AD+BC\right)>{\left(AD+BC\right)}^{2}+{\left(A+B\right)}^{2}\left(CD-E\right). \end{array}$$

In this way, (55) is satisfied; that is, the inequality (45) holds.

In summary, by the biological condition *r*_*B*_ > *δ*_*B*_ + *μ*_*B*_, we find that in polynomial (39), its eigenvalues *λ*_1,2_^2^ = *J*_33_, *λ*_1,3_^2^ = *J*_11_, and *λ*_1,1_^2^ = −*μ*_*C*_ are negative. Additionally, it has also been shown that the four coefficients *a*_1_, *a*_2_, *a*_3_, and *a*_4_ are positive and the two conditions *a*_1_*a*_2_ > *a*_3_ and *a*_1_*a*_2_*a*_3_ > *a*_4_*a*_1_^2^ + *a*_3_^2^ are satisfied when *r*_*B*_^∗^/(*δ*_*B*_^∗^ + *μ*_*B*_^∗^) ≤ *r*_*B*_/(*δ*_*B*_ + *μ*_*B*_) and *r*_*E*_^∗^/*δ*_*E*_^∗^ < *r*_*E*_/*δ*_*E*_ are fulfilled; in particular, *a*_4_ is positive if it also holds that *R*_0_ < 1. Thus, if these three conditions are met: *r*_*B*_^∗^/(*δ*_*B*_^∗^ + *μ*_*B*_^∗^) ≤ *r*_*B*_/(*δ*_*B*_ + *μ*_*B*_), *r*_*E*_^∗^/*δ*_*E*_^∗^ < *r*_*E*_/*δ*_*E*_, and *R*_0_ < 1, then the eigenvalues of the fourth order polynomial in (39) will have a negative real part, and consequently, the point *E*_1_^2^ will be asymptotically stable. On the other hand, by Descartes' rule of signs, if *R*_0_ > 1, then *a*_4_ < 0, and the full polynomial (39) will have a positive eigenvalue, in which case *E*_1_^2^ will be unstable. These results can also be summarized in the following theorem.

**Theorem 8 .**

Assume that the following conditions *r*_*B*_ > *δ*_*B*_ + *μ*_*B*_, *r*_*B*_^∗^/(*δ*_*B*_^∗^ + *μ*_*B*_^∗^) ≤ *r*_*B*_/(*δ*_*B*_ + *μ*_*B*_), and *r*_*E*_^∗^/*δ*_*E*_^∗^ < *r*_*E*_/*δ*_*E*_ are satisfied. The infection-free equilibrium *E*_1_^2^ of system (18) is locally asymptotically stable for *R*_0_ < 1 and unstable for *R*_0_ > 1.

As already mentioned, *E*_1_^2^ is nonhyperbolic when *R*_0_ = 1. It will be shown later that when this happens, a bifurcation occurs.

### 3.2. Global Stability of the Infection-Free Equilibrium

We obtained some conditions on global stability of the infection-free equilibrium of the system (18).

**Theorem 9 .**

Assume that *r*_*B*_ > *δ*_*B*_ + *μ*_*B*_, *r*_*B*_ = *r*_*B*_^∗^, *r*_*E*_ = *r*_*E*_^∗^, *δ*_*B*_ = *δ*_*B*_^∗^, *μ*_*B*_ = *μ*_*B*_^∗^, and *δ*_*E*_^∗^ ≥ *δ*_*E*_. If *R*_0_ ≤ 1, then the infection-free equilibrium *E*_1_^2^ = (*B*_*H*_^∗^, 0, *E*_*H*_^∗^, 0, *C*_*H*_^∗^, 0, 0) of system (18) is globally asymptotically stable in *Ω*_*G*_.

**Proof**

We construct the following Lyapunov function for the system (18):

(62) $$\begin{array}{c} W\left(t\right)=W_{1}\left(t\right)+W_{2}\left(t\right)+W_{3}\left(t\right), \end{array}$$

where the following functions have been defined as

(63) $$\begin{array}{c} W_{1}\left(t\right)=\int_{B_{H}^{*}}^{B_{H}}\left(1-\frac{B_{H}^{*}}{\eta }\right)d\eta +B_{I}+\frac{\beta \sigma \delta_{E}^{*}B_{H}^{*}}{\gamma \mu_{C}^{*}\left(\delta_{E}^{*}-r_{E}\left(1-E_{H}^{*}/K_{E}\right)\right)}E_{I}+\frac{\beta \sigma B_{H}^{*}}{\gamma \mu_{C}^{*}}C_{I}+\frac{\beta B_{H}^{*}}{\gamma }V,\\ W_{2}\left(t\right)=\frac{\beta \sigma \delta_{E}^{*}B_{H}^{*}}{\gamma \mu_{C}^{*}\left(\delta_{E}^{*}-r_{E}\left(1-E_{H}^{*}/K_{E}\right)\right)}\int_{E_{H}^{*}}^{E_{H}}\left(1-\frac{E_{H}^{*}}{\eta }\right)d\eta ,\\ W_{3}\left(t\right)=\frac{\beta \sigma \delta_{E}^{*}B_{H}^{*}}{\gamma \mu_{C}^{*}\left(\delta_{E}^{*}-r_{E}\left(1-E_{H}^{*}/K_{E}\right)\right)}\int_{C_{H}^{*}}^{C_{H}}\left(1-\frac{C_{H}^{*}}{\eta }\right)d\eta . \end{array}$$

The function *W*(*t*) is defined, continuous, and positive definite for all *B*_*H*_, *B*_*I*_, *E*_*H*_, *E*_*I*_, *C*_*H*_, *C*_*I*_, *V* ≥ 0. Also, the global minimum *W*(*B*_*H*_, *B*_*I*_, *E*_*H*_, *E*_*I*_, *C*_*H*_, *C*_*I*_, *V*) = 0 occurs at *E*_1_^2^ = (*B*_*H*_^∗^, 0, *E*_*H*_^∗^, 0, *C*_*H*_^∗^, 0, 0), and therefore, *W* is a Lyapunov function. First, we calculate the time derivative of *W*_1_(*t*).

(64) $$\begin{array}{c} \frac{dW_{1}\left(t\right)}{dt}=\left(1-\frac{B_{H}^{*}}{B_{H}}\right)\frac{dB_{H}}{dt}+\frac{dB_{I}}{dt}+\frac{\beta \sigma \delta_{E}^{*}B_{H}^{*}}{\gamma \mu_{C}^{*}\left(\delta_{E}^{*}-r_{E}\left(1-E_{H}^{*}/K_{E}\right)\right)}\frac{dE_{I}}{dt}+\frac{\beta \sigma B_{H}^{*}}{\gamma \mu_{C}^{*}}\frac{dC_{I}}{dt}+\frac{\beta B_{H}^{*}}{\gamma }\frac{dV}{dt}=\left(1-\frac{B_{H}^{*}}{B_{H}}\right)\left(r_{B}B_{H}\left(1-\frac{B_{H}+B_{I}}{K_{B}}\right)-\left(\delta_{B}+\mu_{B}\right)B_{H}-\beta B_{H}V\right)+r_{B}B_{I}\left(1-\frac{B_{H}+B_{I}}{K_{B}}\right)-\left(\delta_{B}+\mu_{B}\right)B_{I}+\beta B_{H}V+\frac{\beta \sigma \delta_{E}^{*}B_{H}^{*}}{\gamma \mu_{C}^{*}\left(\delta_{E}^{*}-r_{E}\left(1-E_{H}^{*}/K_{E}\right)\right)}\left(\delta_{B}B_{I}+r_{E}E_{I}\left(1-\frac{E_{H}+E_{I}}{K_{E}}\right)-\delta_{E}^{*}E_{I}\right)+\frac{\beta \sigma B_{H}^{*}}{\gamma \mu_{C}^{*}}\left(\delta_{E}^{*}E_{I}-\mu_{C}^{*}C_{I}\right)+\frac{\beta B_{H}^{*}}{\gamma }\left(\sigma C_{I}-\gamma V\right). \end{array}$$

Using *r*_*B*_ − (*δ*_*B*_ + *μ*_*B*_) = (*r*_*B*_/*K*_*B*_)*B*_*H*_^∗^, we have

(65) $$\begin{array}{c} \frac{dW_{1}\left(t\right)}{dt}=-\frac{r_{B}}{K_{B}}\left(B_{H}-B_{H}^{*}\right)\left[\left(B_{H}-B_{H}^{*}\right)+B_{I}\right]-\beta B_{H}V+\beta B_{H}^{*}V+\beta B_{H}V+r_{B}B_{I}\left(1-\frac{B_{H}^{*}}{K_{B}}\right)-\left(\delta_{B}+\mu_{B}\right)B_{I}-\frac{r_{B}}{K_{B}}B_{I}\left[\left(B_{H}-B_{H}^{*}\right)+B_{I}\right]+\frac{\beta \sigma \delta_{E}^{*}B_{H}^{*}}{\gamma \mu_{C}^{*}\left(\delta_{E}^{*}-r_{E}\left(1-E_{H}^{*}/K_{E}\right)\right)}\left[\delta_{B}B_{I}+r_{E}E_{I}\left(1-\frac{E_{H}^{*}}{K_{E}}\right)-\delta_{E}E_{H}-\frac{r_{E}}{K_{E}}E_{I}\left[\left(E_{H}-E_{H}^{*}\right)+E_{I}\right]\right]+\frac{\beta \sigma B_{H}^{*}}{\gamma \mu_{C}^{*}}\left[\delta_{E}^{*}E_{I}-\mu_{C}^{*}C_{I}\right]+\frac{\beta B_{H}^{*}}{\gamma }\left[\sigma C_{I}-\gamma V\right]. \end{array}$$

After several calculations, we have

(66) $$\begin{array}{c} \frac{dW_{1}\left(t\right)}{dt}=-\frac{r_{B}}{K_{B}}{\left[\left(B_{H}-B_{H}^{*}\right)+B_{I}\right]}^{2}-\frac{\beta \sigma \delta_{E}^{*}B_{H}^{*}}{\gamma \mu_{C}^{*}\left(\delta_{E}^{*}-r_{E}\left(1-E_{H}^{*}/K_{E}\right)\right)}\frac{r_{E}}{K_{E}}E_{I}\left[\left(E_{H}-E_{H}^{*}\right)+E_{I}\right]+B_{I}\left[\frac{\beta \sigma \delta_{B}\delta_{E}^{*}B_{H}^{*}}{\gamma \mu_{C}^{*}\left(\delta_{E}^{*}-r_{E}\left(1-E_{H}^{*}/K_{E}\right)\right)}+r_{B}\left(1-\frac{B_{H}^{*}}{K_{B}}\right)-\left(\delta_{B}+\mu_{B}\right)\right]=-\frac{r_{B}}{K_{B}}{\left[\left(B_{H}-B_{H}^{*}\right)+B_{I}\right]}^{2}-\frac{\beta \sigma \delta_{E}^{*}B_{H}^{*}}{\gamma \mu_{C}^{*}\left(\delta_{E}^{*}-r_{E}\left(1-E_{H}^{*}/K_{E}\right)\right)}\frac{r_{E}}{K_{E}}E_{I}\left[\left(E_{H}-E_{H}^{*}\right)+E_{I}\right]-\left(\delta_{B}+\mu_{B}\right)\left(1-R_{0}\right)B_{I}. \end{array}$$

Second, we calculate the time derivative of *W*_2_(*t*).

(67) $$\begin{array}{c} \frac{dW_{2}\left(t\right)}{dt}=\left(1-\frac{E_{H}^{*}}{E_{H}}\right)\frac{dE_{H}}{dt}=\left(1-\frac{E_{H}^{*}}{E_{H}}\right)\left(\delta_{B}B_{H}+r_{E}E_{H}\left(1-\frac{E_{H}+E_{I}}{K_{E}}\right)-\delta_{E}E_{H}\right). \end{array}$$

Considering *r*_*E*_ = (*r*_*E*_/*K*_*E*_)*E*_*H*_^∗^ + *δ*_*E*_ − *δ*_*B*_(*B*_*H*_^∗^/*E*_*H*_^∗^), we obtain

(68) $$\begin{array}{c} \frac{dW_{2}\left(t\right)}{dt}=\frac{\beta \sigma \delta_{B}\delta_{E}^{*}B_{H}^{*}}{\gamma \mu_{C}^{*}\left(\delta_{E}^{*}-r_{E}\left(1-E_{H}^{*}/K_{E}\right)\right)}\frac{r_{E}B_{H}^{*}}{K_{E}}\left(1+\frac{B_{H}^{*}}{B_{H}}-\frac{E_{H}}{E_{H}^{*}}-\frac{B_{H}^{*}E_{H}}{B_{H}E_{H}^{*}}\right)-\frac{\beta \sigma \delta_{E}^{*}B_{H}^{*}}{\gamma \mu_{C}^{*}\left(\delta_{E}^{*}-r_{E}\left(1-E_{H}^{*}/K_{E}\right)\right)}\frac{r_{E}}{K_{E}}\left(E_{H}-E_{H}^{*}\right)\left[\left(E_{H}-E_{H}^{*}\right)+E_{I}\right]=\frac{\beta \sigma \delta_{B}\delta_{E}^{*}B_{H}^{*}}{\gamma \mu_{C}^{*}\left(\delta_{E}^{*}-r_{E}\left(1-E_{H}^{*}/K_{E}\right)\right)}\frac{r_{E}B_{H}^{*}}{K_{E}}\left(3-\frac{B_{H}}{B_{H}^{*}}-\frac{E_{H}}{E_{H}^{*}}-\frac{B_{H}^{*}E_{H}}{B_{H}E_{H}^{*}}\right)+\frac{\beta \sigma \delta_{B}\delta_{E}^{*}B_{H}^{*}}{\gamma \mu_{C}^{*}\left(\delta_{E}^{*}-r_{E}\left(1-E_{H}^{*}/K_{E}\right)\right)}\frac{r_{E}B_{H}^{*}}{K_{E}}\left(\frac{B_{H}^{*}}{B_{H}}+\frac{B_{H}}{B_{H}^{*}}-2\right)-\frac{\beta \sigma \delta_{E}^{*}B_{H}^{*}}{\gamma \mu_{C}^{*}\left(\delta_{E}^{*}-r_{E}\left(1-E_{H}^{*}/K_{E}\right)\right)}\frac{r_{E}}{K_{E}}\left(E_{H}-E_{H}^{*}\right)\left[\left(E_{H}-E_{H}^{*}\right)+E_{I}\right]. \end{array}$$

Writing *βσδ*_*B*_*δ*_*E*_^∗^*B*_*H*_^∗^/(*γμ*_*C*_^∗^(*δ*_*E*_^∗^ − *r*_*E*_(1 − *E*_*H*_^∗^/*K*_*E*_))) in terms of *R*_0_ and considering that *βσδ*_*B*_*δ*_*E*_^∗^*B*_*H*_^∗^/(*γμ*_*C*_^∗^(*δ*_*E*_^∗^ − *r*_*E*_(1 − *E*_*H*_^∗^/*K*_*E*_))) = (*δ*_*B*_ + *μ*_*B*_)(*R*_0_ − (*r*_*B*_/(*δ*_*B*_ + *μ*_*B*_))(1 − *B*_*H*_^∗^/*K*_*B*_)), we find

(69) $$\begin{array}{c} \frac{dW_{2}\left(t\right)}{dt}=\frac{\beta \sigma \delta_{B}\delta_{E}^{*}B_{H}^{*}}{\gamma \mu_{C}^{*}\left(\delta_{E}^{*}-r_{E}\left(1-E_{H}^{*}/K_{E}\right)\right)}\frac{r_{E}B_{H}^{*}}{K_{E}}\left(3-\frac{B_{H}}{B_{H}^{*}}-\frac{E_{H}}{E_{H}^{*}}-\frac{B_{H}^{*}E_{H}}{B_{H}E_{H}^{*}}\right)+\left(R_{0}-\frac{r_{B}}{\delta_{B}+\mu_{B}}\left(1-\frac{B_{H}^{*}}{K_{B}}\right)\right)\frac{\left(\delta_{B}+\mu_{B}\right)r_{E}B_{H}^{*}}{K_{E}}\left(\frac{B_{H}^{*}}{B_{H}}+\frac{B_{H}}{B_{H}^{*}}-2\right)-\frac{\beta \sigma \delta_{E}^{*}B_{H}^{*}}{\gamma \mu_{C}^{*}\left(\delta_{E}^{*}-r_{E}\left(1-E_{H}^{*}/K_{E}\right)\right)}\frac{r_{E}}{K_{E}}\left(E_{H}-E_{H}^{*}\right)\left[\left(E_{H}-E_{H}^{*}\right)+E_{I}\right]=\frac{\beta \sigma \delta_{B}\delta_{E}^{*}B_{H}^{*}}{\gamma \mu_{C}^{*}\left(\delta_{E}^{*}-r_{E}\left(1-E_{H}^{*}/K_{E}\right)\right)}\frac{r_{E}B_{H}^{*}}{K_{E}}\left(3-\frac{B_{H}}{B_{H}^{*}}-\frac{E_{H}}{E_{H}^{*}}-\frac{B_{H}^{*}E_{H}}{B_{H}E_{H}^{*}}\right)+\left(1-R_{0}\right)\frac{\left(\delta_{B}+\mu_{B}\right)r_{E}B_{H}^{*}}{K_{E}}\left(2-\frac{B_{H}^{*}}{B_{H}}-\frac{B_{H}}{B_{H}^{*}}\right)+\left(1-\frac{r_{B}}{\delta_{B}+\mu_{B}}\left(1-\frac{B_{H}^{*}}{K_{B}}\right)\right)\frac{\left(\delta_{B}+\mu_{B}\right)r_{E}B_{H}^{*}}{K_{E}}\left(\frac{B_{H}^{*}}{B_{H}}+\frac{B_{H}}{B_{H}^{*}}-2\right)-\frac{\beta \sigma \delta_{E}^{*}B_{H}^{*}}{\gamma \mu_{C}^{*}\left(\delta_{E}^{*}-r_{E}\left(1-E_{H}^{*}/K_{E}\right)\right)}\frac{r_{E}}{K_{E}}\left(E_{H}-E_{H}^{*}\right)\left[\left(E_{H}-E_{H}^{*}\right)+E_{I}\right]. \end{array}$$

Taking into account that *r*_*B*_(1 − *B*_*H*_^∗^/*K*_*B*_) = *δ*_*B*_ + *μ*_*B*_, we obtain

(70) $$\begin{array}{c} \frac{dW_{2}\left(t\right)}{dt}=\frac{\beta \sigma \delta_{B}\delta_{E}^{*}B_{H}^{*}}{\gamma \mu_{C}^{*}\left(\delta_{E}^{*}-r_{E}\left(1-E_{H}^{*}/K_{E}\right)\right)}\frac{r_{E}B_{H}^{*}}{K_{E}}\left(3-\frac{B_{H}}{B_{H}^{*}}-\frac{E_{H}}{E_{H}^{*}}-\frac{B_{H}^{*}E_{H}}{B_{H}E_{H}^{*}}\right)+\left(1-R_{0}\right)\frac{\left(\delta_{B}+\mu_{B}\right)r_{E}B_{H}^{*}}{K_{E}}\left(2-\frac{B_{H}^{*}}{B_{H}}-\frac{B_{H}}{B_{H}^{*}}\right)-\frac{\beta \sigma \delta_{E}^{*}B_{H}^{*}}{\gamma \mu_{C}^{*}\left(\delta_{E}^{*}-r_{E}\left(1-E_{H}^{*}/K_{E}\right)\right)}\frac{r_{E}}{K_{E}}\left(E_{H}-E_{H}^{*}\right)\left[\left(E_{H}-E_{H}^{*}\right)+E_{I}\right]. \end{array}$$

Third, we calculate the time derivative of *W*_3_(*t*).

(71) $$\begin{array}{c} \frac{dW_{3}\left(t\right)}{dt}=\left(1-\frac{C_{H}^{*}}{C_{H}}\right)\frac{dC_{H}}{dt}=\left(1-\frac{C_{H}^{*}}{C_{H}}\right)\left(\delta_{E}E_{H}-\mu_{C}C_{H}\right). \end{array}$$

Using *δ*_*E*_*E*_*H*_^∗^ = *μ*_*C*_*C*_*H*_^∗^, we have

(72) $$\begin{array}{c} \frac{dW_{3}\left(t\right)}{dt}=\frac{\beta \sigma \delta_{E}^{*}B_{H}^{*}}{\gamma \mu_{C}^{*}\left(\delta_{E}^{*}-r_{E}\left(1-E_{H}^{*}/K_{E}\right)\right)}\delta_{E}E_{H}^{*}\left(\frac{E_{H}}{E_{H}^{*}}-\frac{C_{H}}{C_{H}^{*}}-\frac{E_{H}C_{H}^{*}}{E_{H}^{*}C_{H}}+1\right)=\frac{\beta \sigma \delta_{E}^{*}B_{H}^{*}}{\gamma \mu_{C}^{*}\left(\delta_{E}^{*}-r_{E}\left(1-E_{H}^{*}/K_{E}\right)\right)}\delta_{E}E_{H}^{*}\left(3-\frac{E_{H}^{*}}{E_{H}}-\frac{C_{H}}{C_{H}^{*}}-\frac{E_{H}C_{H}^{*}}{E_{H}^{*}C_{H}}\right)+\frac{\beta \sigma \delta_{E}^{*}B_{H}^{*}}{\gamma \mu_{C}^{*}\left(\delta_{E}^{*}-r_{E}\left(1-E_{H}^{*}/K_{E}\right)\right)}\delta_{E}E_{H}^{*}\left(\frac{E_{H}}{E_{H}^{*}}+\frac{E_{H}^{*}}{E_{H}}-2\right),=\frac{\beta \sigma \delta_{E}^{*}B_{H}^{*}}{\gamma \mu_{C}^{*}\left(\delta_{E}^{*}-r_{E}\left(1-E_{H}^{*}/K_{E}\right)\right)}\delta_{E}E_{H}^{*}\left(3-\frac{E_{H}^{*}}{E_{H}}-\frac{C_{H}}{C_{H}^{*}}-\frac{E_{H}C_{H}^{*}}{E_{H}^{*}C_{H}}\right)+\left(R_{0}-\frac{r_{B}}{\delta_{B}+\mu_{B}}\left(1-\frac{B_{H}^{*}}{K_{B}}\right)\right)\frac{\delta_{E}\left(\delta_{B}+\mu_{B}\right)E_{H}^{*}}{\delta_{B}}\left(\frac{E_{H}}{E_{H}^{*}}+\frac{E_{H}^{*}}{E_{H}}-2\right)=\frac{\beta \sigma \delta_{E}^{*}B_{H}^{*}}{\gamma \mu_{C}^{*}\left(\delta_{E}^{*}-r_{E}\left(1-E_{H}^{*}/K_{E}\right)\right)}\delta_{E}E_{H}^{*}\left(3-\frac{E_{H}^{*}}{E_{H}}-\frac{C_{H}}{C_{H}^{*}}-\frac{E_{H}C_{H}^{*}}{E_{H}^{*}C_{H}}\right)+\left(1-R_{0}\right)\frac{\delta_{E}\left(\delta_{B}+\mu_{B}\right)E_{H}^{*}}{\delta_{B}}\left(2-\frac{E_{H}}{E_{H}^{*}}-\frac{E_{H}^{*}}{E_{H}}\right)+\left(\frac{r_{B}}{\delta_{B}+\mu_{B}}\left(1-\frac{B_{H}^{*}}{K_{B}}\right)-1\right)\frac{\delta_{E}\left(\delta_{B}+\mu_{B}\right)E_{H}^{*}}{\delta_{B}}\left(2-\frac{E_{H}}{E_{H}^{*}}-\frac{E_{H}^{*}}{E_{H}}\right). \end{array}$$

Considering *r*_*B*_(1 − *B*_*H*_^∗^/*K*_*B*_) = *δ*_*B*_ + *μ*_*B*_, we find

(73) $$\begin{array}{c} \frac{dW_{3}\left(t\right)}{dt}=\frac{\beta \sigma \delta_{E}^{*}B_{H}^{*}}{\gamma \mu_{C}^{*}\left(\delta_{E}^{*}-r_{E}\left(1-E_{H}^{*}/K_{E}\right)\right)}\delta_{E}E_{H}^{*}\left(3-\frac{E_{H}^{*}}{E_{H}}-\frac{C_{H}}{C_{H}^{*}}-\frac{E_{H}C_{H}^{*}}{E_{H}^{*}C_{H}}\right)+\left(1-R_{0}\right)\frac{\delta_{E}\left(\delta_{B}+\mu_{B}\right)E_{H}^{*}}{\delta_{B}}\left(2-\frac{E_{H}}{E_{H}^{*}}-\frac{E_{H}^{*}}{E_{H}}\right). \end{array}$$

Finally, considering expressions (66), (70), and (73), we obtain

(74) $$\begin{array}{c} \frac{dW\left(t\right)}{dt}=\frac{dW_{1}\left(t\right)}{dt}+\frac{dW_{2}\left(t\right)}{dt}+\frac{dW_{3}\left(t\right)}{dt}=-\frac{r_{B}}{K_{B}}{\left[\left(B_{H}-B_{H}^{*}\right)+B_{I}\right]}^{2}-\frac{\beta \sigma \delta_{E}^{*}B_{H}^{*}}{\gamma \mu_{C}^{*}\left(\delta_{E}^{*}-r_{E}\left(1-E_{H}^{*}/K_{E}\right)\right)}\frac{r_{E}}{K_{E}}{\left[\left(E_{H}-E_{H}^{*}\right)+E_{I}\right]}^{2}-\left(\delta_{B}+\mu_{B}\right)\left(1-R_{0}\right)B_{I}+\frac{\beta \sigma \delta_{B}\delta_{E}^{*}B_{H}^{*}}{\gamma \mu_{C}^{*}\left(\delta_{E}^{*}-r_{E}\left(1-E_{H}^{*}/K_{E}\right)\right)}\frac{r_{E}B_{H}^{*}}{K_{E}}\left(3-\frac{B_{H}}{B_{H}^{*}}-\frac{E_{H}}{E_{H}^{*}}-\frac{B_{H}^{*}E_{H}}{B_{H}E_{H}^{*}}\right)+\left(1-R_{0}\right)\frac{\left(\delta_{B}+\mu_{B}\right)r_{E}B_{H}^{*}}{K_{E}}\left(2-\frac{B_{H}^{*}}{B_{H}}-\frac{B_{H}}{B_{H}^{*}}\right)+\frac{\beta \sigma \delta_{E}^{*}B_{H}^{*}}{\gamma \mu_{C}^{*}\left(\delta_{E}^{*}-r_{E}\left(1-E_{H}^{*}/K_{E}\right)\right)}\delta_{E}E_{H}^{*}\left(3-\frac{E_{H}^{*}}{E_{H}}-\frac{C_{H}}{C_{H}^{*}}-\frac{E_{H}C_{H}^{*}}{E_{H}^{*}C_{H}}\right)+\left(1-R_{0}\right)\frac{\delta_{E}\left(\delta_{B}+\mu_{B}\right)E_{H}^{*}}{\delta_{B}}\left(2-\frac{E_{H}}{E_{H}^{*}}-\frac{E_{H}^{*}}{E_{H}}\right). \end{array}$$

If *R*_0_ ≤ 1, then *dW*/*dt* ≤ 0. Note that *dW*/*dt* = 0 if and only if *B*_*H*_ = *B*_*H*_^∗^, *B*_*I*_ = 0, *E*_*H*_ = *E*_*H*_^∗^, and *E*_*I*_ = 0 or *R*_0_ = 1, *B*_*H*_ = *B*_*H*_^∗^, *B*_*I*_ = 0, *E*_*H*_ = *E*_*H*_^∗^, and *E*_*I*_ = 0. Therefore, the largest compact invariant set in {(*B*_*H*_(*t*), *B*_*I*_(*t*), *E*_*H*_(*t*), *E*_*I*_(*t*), *C*_*H*_(*t*), *C*_*I*_(*t*), *V*(*t*)): *dW*/*dt* = 0} is the singleton {*E*_1_^2^}. By the classical LaSalle invariance principle (Theorem 5.3 of [30]), *E*_1_^2^ is globally asymptotically stable in *Ω*_*G*_ if *R*_0_ ≤ 1.

### 3.3. Existence of a Forward or Backward Bifurcation

It has already been mentioned that when *R*_0_ = 1, in the characteristic equation (39), *a*_4_ vanishes given rise to a zero eigenvalue and the infection-free equilibrium point *E*_1_^2^ is nonhyperbolic. This suggests that in this case, a bifurcation occurs at that point. Indeed, this happens, as we will show below. For this purpose, we will use the Theorem 4.1 of [31]. According to this result, it is required to rewrite system (18) as

(75) $$\begin{array}{c} \frac{dx_{1}}{dt}=a_{0}x_{1}-b_{0}x_{1}x_{2}-\beta x_{1}x_{7}-b_{0}x_{1}^{2}\equiv f_{1},\\ \frac{dx_{2}}{dt}=a_{1}x_{2}-b_{1}x_{1}x_{2}+\beta x_{1}x_{7}-b_{1}x_{2}^{2}\equiv f_{2},\\ \frac{dx_{3}}{dt}=\delta_{B}x_{1}+c_{0}x_{3}-d_{0}x_{3}x_{4}-d_{0}x_{3}^{2}\equiv f_{3},\\ \frac{dx_{4}}{dt}=x_{2}\delta_{B}^{*}+c_{1}x_{4}-d_{1}x_{3}x_{4}-d_{1}x_{4}^{2}\equiv f_{4},\\ \frac{dx_{5}}{dt}=\delta_{E}x_{3}-\mu_{C}x_{5}\equiv f_{5},\\ \frac{dx_{6}}{dt}=\delta_{E}^{*}x_{4}-\mu_{C}^{*}x_{6}\equiv f_{6},\\ \frac{dx_{7}}{dt}=\sigma x_{6}-\gamma x_{7}\equiv f_{7}, \end{array}$$

which is in terms of the new variables

(76) $$\begin{array}{c} x_{1}\equiv B_{H},\;x_{2}\equiv B_{I},\;x_{3}\equiv E_{H},\;x_{4}\equiv E_{I},\;x_{5}\equiv C_{H},\;x_{6}\equiv C_{I},\;x_{7}\equiv V, \end{array}$$

and the new parameters

(77) $$\begin{array}{c} a_{0}\equiv r_{B}-\delta_{B}-\mu_{B},\;a_{1}\equiv r_{B}^{*}-\delta_{B}^{*}-\mu_{B}^{*},\;b_{0}\equiv \frac{r_{B}}{K_{B}},\;b_{1}\equiv \frac{r_{B}^{*}}{K_{B}},\\ c_{0}\equiv r_{E}-\delta_{E},\;c_{1}\equiv r_{E}^{*}-\delta_{E}^{*},\;d_{0}\equiv \frac{r_{E}}{K_{E}},\;d_{1}\equiv \frac{r_{E}^{*}}{K_{E}}. \end{array}$$

We will consider that *β* is the bifurcation parameter and that when *R*_0_ = 1, according to definition of *R*_0_, this parameter takes the value

(78) $$\begin{array}{c} \beta^{*}=\frac{\gamma \mu_{C}^{*}J_{22}J_{44}}{\sigma \delta_{B}^{*}\delta_{E}^{*}x_{1}^{*}}. \end{array}$$

The Jacobian matrix of system (75) evaluated at the equilibrium point *E*_1_^2^, when *β* = *β*^∗^, is

(79) $$\begin{array}{c} J\left(E_{1}^{2}\right)=\left(\begin{array}{ccccccc} J_{11} & -b_{0}x_{1}^{*} & 0 & 0 & 0 & 0 & -\beta^{*}x_{1}^{*}\\ 0 & J_{22} & 0 & 0 & 0 & 0 & \beta^{*}x_{1}^{*}\\ \delta_{B} & 0 & J_{33} & -d_{0}x_{3}^{*} & 0 & 0 & 0\\ 0 & \delta_{B}^{*} & 0 & J_{44} & 0 & 0 & 0\\ 0 & 0 & \delta_{E} & 0 & -\mu_{C} & 0 & 0\\ 0 & 0 & 0 & \delta_{E}^{*} & 0 & -\mu_{C}^{*} & 0\\ 0 & 0 & 0 & 0 & 0 & \sigma & -\gamma \end{array}\right), \end{array}$$

where the quantities *J*_11_, *J*_22_, *J*_33_, and *J*_44_, given by (33)–(36), are written as

(80) $$\begin{array}{c} J_{11}=a_{0}-2b_{0}x_{1}^{*},J_{22}=a_{1}-b_{1}x_{1}^{*},J_{33}=c_{0}-2d_{0}x_{3}^{*},J_{44}=c_{1}-d_{1}x_{3}^{*}. \end{array}$$

In this case, we know that zero is a simple eigenvalue of (79). A right eigenvector associated with zero eigenvalue is

(81) $$\begin{array}{c} w=\frac{1}{\left(\mu_{C}^{*}+\gamma \right)J_{44}J_{22}-\gamma \mu_{C}^{*}\left(J_{22}+J_{44}\right)}\left(\begin{array}{c} \frac{\gamma \mu_{C}^{*}J_{44}}{\sigma \delta_{B}^{*}\delta_{E}^{*}J_{11}}\left(J_{22}-b_{0}x_{1}^{*}\right)\\ -\frac{J_{44}}{\delta_{B}^{*}}\frac{\mu_{C}^{*}}{\delta_{E}^{*}}\frac{\gamma }{\sigma }\\ \frac{\gamma \mu_{C}^{*}}{\sigma \delta_{B}^{*}\delta_{E}^{*}}\left[-\frac{\delta_{B}J_{44}}{J_{11}J_{33}}\left(J_{22}-b_{0}x_{1}^{*}\right)+\frac{\delta_{B}^{*}d_{0}x_{3}^{*}}{J_{33}}\right]\\ \frac{\mu_{C}^{*}}{\delta_{E}^{*}}\frac{\gamma }{\sigma }\\ \frac{\delta_{E}}{\mu_{C}}\frac{\gamma \mu_{C}^{*}}{\sigma \delta_{B}^{*}\delta_{E}^{*}}\left[-\frac{\delta_{B}J_{44}}{J_{11}J_{33}}\left(J_{22}-b_{0}x_{1}^{*}\right)+\frac{\delta_{B}^{*}d_{0}x_{3}^{*}}{J_{33}}\right]\\ \frac{\gamma }{\sigma }\\ 1 \end{array}\right), \end{array}$$

and the left eigenvector *v*, satisfying *v* · *w* = 1, is

(82) $$\begin{array}{c} v^{T}=\sigma \delta_{B}^{*}\delta_{E}^{*}\left(\begin{array}{c} 0\\ 1\\ 0\\ -\frac{J_{22}}{\delta_{B}^{*}}\\ 0\\ \frac{\beta^{*}\sigma x_{1}^{*}}{\gamma \mu_{C}^{*}}\\ \frac{\beta^{*}x_{1}^{*}}{\gamma } \end{array}\right). \end{array}$$

By algebraic calculations, it can be shown that the required nonzero second-order partial derivatives evaluated at *E*_1_^2^, which are contained in the quantities *a* and *b* given in Theorem 4.1 of [31], are

(83) $$\begin{array}{c} \frac{\partial^{2}f_{2}\left(E_{1}^{2}\right)}{\partial x_{1}\partial x_{2}}=\frac{\partial^{2}f_{2}\left(E_{1}^{2}\right)}{\partial x_{2}\partial x_{1}}=-b_{1},\frac{\partial^{2}f_{2}\left(E_{1}^{2}\right)}{\partial x_{1}\partial x_{7}}=\frac{\partial^{2}f_{2}\left(E_{1}^{2}\right)}{\partial x_{7}\partial x_{1}}=\beta^{*},\frac{\partial^{2}f_{2}\left(E_{1}^{2}\right)}{\partial x_{2}\partial x_{2}}=-2b_{1},\\ \frac{\partial^{2}f_{4}\left(E_{1}^{2}\right)}{\partial x_{3}\partial x_{4}}=\frac{\partial^{2}f_{4}\left(E_{1}^{2}\right)}{\partial x_{4}\partial x_{3}}=-d_{1},\frac{\partial^{2}f_{4}\left(E_{1}^{2}\right)}{\partial x_{4}\partial x_{4}}=-2d_{1},\\ \frac{\partial^{2}f_{2}\left(E_{1}^{2}\right)}{\partial \beta \partial x_{7}}=\frac{\partial^{2}f_{2}\left(E_{1}^{2}\right)}{\partial x_{7}\partial \beta }=x_{1}^{*}. \end{array}$$

Thus, the quantities *a* and *b* take the form

(84) $$\begin{array}{c} a=2\beta^{*}v_{2}w_{1}w_{7}-2b_{1}v_{2}w_{2}\left(w_{1}+w_{2}\right)-2d_{1}v_{4}w_{4}\left(w_{3}+w_{4}\right), \end{array}$$

(85) $$\begin{array}{c} b=v_{2}w_{7}x_{1}^{*}, \end{array}$$

where *w*_1_, *w*_2_, *w*_3_, *w*_4_, and *w*_7_ are the first, second, third, fourth, and seventh components of eigenvector (81), while *v*_2_ is the second component of left eigenvector (82). Given that in (84) the first term on the right hand side of equality depends on *β*^∗^, the relationship that it has with the other terms will determine whether *a* > 0 or *a* < 0. On the other hand, *b* > 0 since *v*_2_ > 0, *w*_7_ > 0, and *x*_1_^∗^ > 0. Therefore, taking into account the above and Theorem 4.1 of [31], the following theorem can be established.

**Theorem 10 .**

The infection-free equilibrium point *E*_1_^2^, when *R*_0_ = 1, presents a backward bifurcation if *β*^∗^ < *β*_*R*_, while it has a forward bifurcation if *β*^∗^ > *β*_*R*_, where

(86) $$\begin{array}{c} \beta_{R}\equiv b_{1}\frac{v_{2}w_{2}\left(w_{1}+w_{2}\right)}{v_{2}w_{1}w_{7}}+d_{1}\frac{v_{4}w_{4}\left(w_{3}+w_{4}\right)}{v_{2}w_{1}w_{7}}. \end{array}$$

It is important to note that, as a consequence of the previous result, when *R*_0_ > 1, there is a family of asymptotically stable infected equilibrium points, which we will denote as $E_{2}^{2}=\left({\bar{B}}_{H},{\bar{B}}_{I},{\bar{E}}_{H},{\bar{E}}_{I},{\bar{C}}_{H},{\bar{C}}_{I},\bar{V}\right)$, constituting the upper branch of these types of bifurcations.

## 4. Viral Kinetic *In Silico*

In this section, the typical values of all the parameters involved in the HPV viral dynamics model given by the system (18) are indicated. With these values, three relevant features of this model are determined numerically. The first one is the type of local bifurcation that this system exhibits when *R*_0_ = 1 at the infection-free equilibrium point *E*_1_^2^. The second is the determination, when *R*_0_ > 1, of the regions of existence and stability of the infected equilibrium point *E*_2_^2^. The third consists of the simulation of different scenarios of interest, such as the transient, acute, latent, and chronic infections visualized in Figure 2.

### 4.1. Typical Parameters of the HPV Viral Dynamics Model

Most of the parameter values were obtained from the literature (see Table 1). The initial conditions of the number of cells in each stratum were calculated from the cell count in the micrographs of Figure 2 in Walker et al. [32]. We present simulations on a rectangular area of 2585288 *μ*m^2^ of epithelial tissue, where the length is 7282.5 *μm* and the height is 355 *μm*. We estimate *K*_*B*_ and *K*_*E*_ assuming that the tissue is divided into four equal parts, all having the same area, and each is divided by the area that a cell occupies according to its stratum. Consequently, the initial conditions of the viral kinetic *in silico* are the following: *B*_*H*_(0) = 1000, *B*_*I*_(0) = *E*_*I*_(0) = *C*_*I*_(0) = 0, *E*_*H*_(0) = 617, *C*_*H*_(0) = 226, and *V*(0) = 100. For parameters *r*_*B*_^∗^ and *r*_*E*_^∗^, they were proposed with values close to the proliferation rates of uninfected stratum basale and stratum intermedium cells, respectively.

### 4.2. Existence of a Forward Bifurcation at Infection-Free Equilibrium Point

To determine the type of bifurcation that occurs, when *R*_0_ = 1, at the equilibrium point *E*_1_^2^, were considered *β* = 10^−6^, *σ* = 10^3^ and all other required quantities from Table 1. With these values it is found, by (85), that *b* = 152,994, which is positive. Furthermore, it is found, according to (78) and (86), respectively, that *β*^∗^ = 9.941 × 10^−8^ and *β*_*R*_ = 4.351 × 10^−8^. Since for the typical values of the parameters considered, we find that *β*^∗^ > *β*_*R*_; consequently, according to Theorem 13, at the infection-free equilibrium point *E*_1_^2^, when *R*_0_ = 1, there is a forward bifurcation.

### 4.3. Regions of Existence and Stability of the Infected Equilibrium Point

A numerical scheme was implemented to show the regions of existence and local stability of the infected equilibrium point *E*_2_^2^ of the model (18) when *R*_0_ is greater to unity. All of the parameters were set, except the rate of viral transmission *β* and the production rate of free virions *σ*. Because an infected cell produces up to 1000 viral particles [11], we take this restriction for the choice of the parameter space *σ*. For each ordered pair (*σ*, *β*), we determine numerically the basic reproductive number value and the coordinate $\bar{V}$ of the infected equilibrium point *E*_2_^2^ using the *bisection method*. We calculate the eigenvalues of the Jacobian matrix (22) evaluated at *E*_2_^2^ using the *eig* function in MATLAB [35], and the signs of the real part of the eigenvalues were identified for the stability classification of the hyperbolic equilibrium point.

The regions of existence and stability of the infected equilibrium point are shown in Figure 5, given the parameters *σ* and *β*. The green, blue, and red regions represent the values of both parameters that make *E*_2_^2^ not exist, or be locally asymptotically stable or unstable, respectively.

### 4.4. Simulation of Different Scenarios of Interest

When some HPV genotype is in a host, there is no infection in the cells of the stratum basale and the viral load is removed until its complete elimination during the following days, without altering the homeostasis of the epithelium. Similar dynamics are consistent with transient type infections. *σ* = 1000 and *β* = 9.447 × 10^−8^ such that *R*_0_ < 1 in this scenario is shown in Figure 6. In this case, the infection-free equilibrium point is locally asymptotically stable.

Some infections successfully establish, replicate the viral genome, produce viral particles, and are eventually cleared. This kinetics is known as acute infection.  Figure 7 with *σ* = 1000 and *β* = 8.390 × 10^−4^ such that *R*_0_ > 1 shows that a (*σ*, *β*) belongs to the instability region of *E*_1_^2^ and to the asymptotically stable region of *E*_2_^2^, as shown in Figure 5. In this scenario, the homeostasis of the epithelial cells is altered, and the viral load describes a unimodal curve for 1500 days, and finally, the infection is resolved.

Latent infections are another form of kinetics, where the acute infections only appear to clear, but the viral genome remains in the infected cell without detectable activity. This is illustrated in Figure 8 with *σ* = 1000 and *β* = 7.247 × 10^−7^ and Figure 9 with *σ* = 1000 and *β* = 2.155 × 10^−6^ such that *R*_0_ > 1. The ordered pair (*σ*, *β*) for Figure 8 belongs to the region of asymptotic stability of *E*_2_^2^ of Figure 5 and (*σ*, *β*) for Figure 9 belongs to the region of instability of *E*_2_^2^ of Figure 5. According to Figure 8, a rapid growth of viral load is shown but without completely infecting the epithelium during the first 250 days after infection. After this period, the viral load tends to decrease up to 1000 days postinfection. From this time on, the dynamics show a similar pattern, which is comparable with damped dynamics until the infection is stabilized throughout the epithelium. This behavior shows the dynamics of a latent infection that can turn into a chronic infection. Likewise, Figure 9 shows the rapid growth of viral load during the first 100 days and decreases until about 2000 days after infection. Although a similar pattern holds over time, the solution does not show damped dynamics as in Figure 8. In this scenario, the resolution of the infection does not occur because the model (18) does not consider mechanisms of prevention or elimination of the virus, the epithelium in its entirety is infected rapidly, and there can be no proliferation of healthy basal cells.

Chronic infections are acute infections that not cleared and maintain viral activity over time. This is shown in Figure 10 with *σ* = 1000 and *β* = 1.447 × 10^−7^ such that *R*_0_ > 1. The ordered pair (*σ*, *β*) belongs to the region of asymptotic stability of *E*_2_^2^ of Figure 5. After infection of the epithelium, viral load production increases monotonically during the first 1500 days until equilibrium is reached, but the infection of the cells does not occur in all stratified epithelial tissue.

## 5. Local Sensitivity Analysis

In the context of viral infections, sensitivity analysis can provide valuable information on how HPV viral kinetics are with respect to changes in model parameters. Local sensitivity analysis is a classic method that studies the impact of small perturbations on the model outputs. The normalized forward sensitivity index of a variable, *u*, that depends differentiable on a parameter, *p*, is defined as

(87) $$\begin{array}{c} \Psi_{p}^{u}=\frac{p}{u}\frac{\partial u}{\partial p}. \end{array}$$

Local sensitivity analysis is carried out in order to identify which parameters have the greatest influence on changes in the values of *R*_0_. As we have an explicit formula for *R*_0_, we derive an analytical expression for the sensitivity of *R*_0_,

(88) $$\begin{array}{c} \Psi_{p}^{R_{0}}=\frac{p}{R_{0}}\frac{\partial R_{0}}{\partial p}, \end{array}$$

to each of the parameters described in *R*_0_.

Figure 11 shows that all the parameters have either positive or negative effects on the *R*_0_. According to the sensitivity indices illustrated in Figure 11, we observe that the parameters, namely, *r*_*E*_^∗^, *β*, *σ*, and *δ*_*E*_^∗^, are the most positively sensitive parameters, respectively. This implies that decreasing the values of these parameters will decrease *R*_0_. Parameters *μ*_*C*_^∗^, *δ*_*B*_, *δ*_*B*_^∗^, and *γ* are the most negatively sensitive parameters. This implies that increasing the values of these parameters will decrease *R*_0_.

## 6. Discussion

Several approaches have been reported in the literature for the mathematical modeling of the process of viral infection by HPV. For example, Verma et al. [24] proposed a model of HIV/HPV coinfection in oral mucosal epithelial cells with anti-HPV immune response. They consider the basal and suprabasal layers of oral mucosal but ignore viral transmission via suprabasal differentiation, which is very relevant in the persistence of the virus. In their simulations, the authors reproduce acute and chronic infections. Murall et al. [25] developed a viral dynamics model of the cervical stratified epithelium of cornified, granular, spinous, and basal layers. In their simulations, they reproduce a scenario where the infection is inoculated with a few cells and the microabrasion repairs quickly, and another scenario of slow growing HR HPV infection that spontaneously regresses. However, this model ignores the epithelial cellular dynamics of healthy tissue, and it models the viral transmission via suprabasal differentiation with a linear term. Motivated by this review, we proposed a mathematical model that includes several layers of the healthy and infected squamous epithelium without the presence of the immune response. We modeled the viral transmission via suprabasal differentiation with a full logistic term.

We start by proposing a model of the epithelial cellular dynamics of the cervix stratified epithelium of three (basale, intermedium, and corneum) stratums, given by the system (1), where the stratum intermedium is formed by granular and spinous layers. This assumption considers that the dynamics of basal and suprabasal differentiation are homogeneous between the two stratums. In addition, we have a simpler mathematical model that is easier to deal with from qualitative analysis. We determine biological condition *r*_*B*_ > *δ*_*B*_ + *μ*_*B*_ for the existence of the epithelial cell homeostasis equilibrium *E*_1_^1^ = (*B*_*H*_^∗^, *E*_*H*_^∗^, *C*_*H*_^∗^), and consequently, we include cellular dynamics of the cervical epithelium. We have proven that trivial equilibrium *E*_0_^1^ = (0, 0, 0) always exists and is unstable. Using the method of Lyapunov functions and a theorem on limiting systems, we have proven that the epithelial cell homeostasis equilibrium is globally asymptotically stable when the biological condition is satisfied.

Later, we formulated an extended model, given by system (18), in which the infection by the HPV virus was taken into account. For this system, the basic reproductive number *R*_0_ of the infection was calculated. This allowed us to design the different scenarios of the theoretical viral loads. The model also has a trivial equilibrium point *E*_0_^2^ and an epithelial cell homeostasis one *E*_1_^2^. It was proved that *E*_0_^2^ always exists and is unstable, whereas if the biological condition *r*_*B*_ > *δ*_*B*_ + *μ*_*B*_ is satisfied, then *E*_1_^2^ exists. If the following conditions *r*_*B*_^∗^/(*δ*_*B*_^∗^ + *μ*_*B*_^∗^) ≤ *r*_*B*_/(*δ*_*B*_ + *μ*_*B*_) and *r*_*E*_^∗^/*δ*_*E*_^∗^ < *r*_*E*_/*δ*_*E*_ are satisfied, the *E*_1_^2^ is locally asymptotically stable if *R*_0_ < 1 and unstable when *R*_0_ > 1. We note that the stability conditions have the following biological interpretation: *r*_*E*_^∗^/*δ*_*E*_^∗^ < *r*_*E*_/*δ*_*E*_, the ratio of proliferation rate and differentiation rate of the infected stratum intermedium cell is less than ratio of proliferation rate and differentiation rate of the uninfected stratum intermedium cells. A similar interpretation can be made of the condition *r*_*B*_^∗^/(*δ*_*B*_^∗^ + *μ*_*B*_^∗^) ≤ *r*_*B*_/(*δ*_*B*_ + *μ*_*B*_). Using an elegant construction of a Lyapunov function, we obtained conditions on parameters (*r*_*B*_ = *r*_*B*_^∗^, *r*_*E*_ = *r*_*E*_^∗^, *δ*_*B*_ = *δ*_*B*_^∗^, *μ*_*B*_ = *μ*_*B*_^∗^, and *δ*_*E*_^∗^ ≥ *δ*_*E*_) to prove the global asymptotic stability of the epithelial cell homeostasis equilibrium. We observe that under the following conditions on the parameters *r*_*B*_ = *r*_*B*_^∗^, *r*_*E*_ = *r*_*E*_^∗^, *δ*_*B*_ = *δ*_*B*_^∗^, *μ*_*B*_ = *μ*_*B*_^∗^, and *δ*_*E*_^∗^ > *δ*_*E*_, the conditions of the Theorem 11 continue to be satisfied. Furthermore, it was shown that when *R*_0_ = 1, *E*_1_^2^ is nonhyperbolic and that in this case, it experiences a forward bifurcation. This last result shows the existence of a family of asymptotically stable infected equilibrium points, denoted as *E*_2_^2^, which bifurcate from the nonhyperbolic equilibrium point and are located in the upper branch of the forward bifurcation.

We numerically study the local stability of the infected equilibrium *E*_2_^2^ varying the virus-to-cell transmission rate and the viral production rate, and we obtained the regions of stability that are shown in Figure 5. We have reproduced the viral kinetics *in silico* that have been proposed by Alizon et al. [12] as the transient, acute, latent, and chronic infections. In the transient infection (Figure 6), the viral load is removed until its complete elimination during the following days, without altering the homeostasis of the epithelium. In acute infection, the viral load describes a unimodal curve for fifteen hundred days, and the homeostasis of the epithelial cells is altered; finally, the infection is resolved (Figure 7). In latent infection, the viral load shows behavior of damped and self-sustaining oscillations (Figures 8 and 9), and the resolution of the infection does not occur, and the epithelium in its entirety is infected rapidly. In the chronic infection, the viral load production increases monotonically during the first thousand days until equilibrium is reached, but the infection of the cells does not occur in all stratified epithelial tissue (Figure 10). All of the simulations were performed with the initial condition of viral inoculation of *V*(0) = 100. We also performed simulations with different initial values in *V*(0), specifically with *V*(0) = 10 and *V*(0) = 1000, and we obtained the same scenarios for each case.

As described by Alizon et al. [12], transient, acute, latent, and chronic infections differ in terms of viral activity, such as viral and cellular gene expression patterns, effects on cell replication dynamics, or induced local immunosuppression. Currently, protocols are being developed, such as the PAPCLEAR study [15], that allow adequate monitoring to characterize the stages of infection in healthy young women, particularly in the detection of viral genetic material associated with latent or chronic infections. The PAPCLEAR study will be relevant because of its impact in understanding the natural history of cervical HPV infections as the possible integration of longitudinal data to mathematical models.

Sensitivity analysis provides insights on possible strategies for the control of a viral infection. The results of the local sensitivity analysis (Figure 11) should be considered together with simulated outputs of virus dynamics models and the possible interventions to be carried out. In our model of the dynamics of HPV infection, the viral transmission rate (*β*) and viral production rate (*σ*) could be reduced by developing antiviral therapies targeting inhibition of new infections and viral replication, respectively, which is still under investigation [36, 37]. The viral clearance rate (*γ*) is traditionally increased by the antibody immune response induced by vaccines. Vaccine-induced antibody levels have been reported to be stable over time, which is associated with high long-term protection [38]. Differentiation rate of infected basal cell (*δ*_*B*_^∗^) could be decreased by cytotoxic T cell immune response, but there is no direct evidence that viral antigen-specific immune effector mechanisms are responsible for virus elimination [39].

Our model (18) suffers from a limitation because it does not consider the four strata of the stratified epithelium, but the model illustrates all the theoretical viral kinetic scenarios proposed by Alizon et al. [12]. Therefore, the innate and cellular immune response can be studied in the future work where it is possible to reproduce the kinetics obtained in the retrospective study [13] as the kinetics of latency with regression or progression of the infection.

## 7. Conclusions

In summary, in this research work, the dynamics of an HPV model were studied through the use of qualitative and numerical analyses. Regarding the first, the positivity and boundary conditions of their solutions were determined, and their main equilibrium points were found, as well as their local and global stabilities. In addition, it was shown that, when *R*_0_ = 1, the model has a nonhyperbolic equilibrium point which, for typical values of the parameters involved, gives rise to a forward bifurcation; consequently, there is a family of asymptotically stable infected equilibrium points *E*_2_^2^ that branch off from the nonhyperbolic point. It is worth mentioning that this last result is merely local and only valid in the neighborhood of *R*_0_ = 1, so the qualitative analysis of the local and global stabilities of these points for values of *R*_0_ much greater than one is still an open problem.

Through numerical analysis of the model solutions, we study some features of the intricate behavior that they exhibit around the infected equilibrium point *E*_2_^2^. Specifically, our simulated results (i.e., viral kinetic *in silico*) suggested that the dynamics of HPV model reproduce the transient, acute, latent, and chronic infections that have been reported in studies of the natural history of HPV.

Finally, using local sensitivity analysis, we found some parameters that could be controlled to remove HPV infection in epithelial tissue, as the viral transmission rate (*β*), viral production rate (*σ*), and viral clearance rate (*γ*).

## Figures and Tables

**Figure 1:** Cervical stratified squamous epithelial cell architecture.

**Figure 2:** Theoretical HPV viral load kinetics. Figure adapted from Alizon et al. [12].

**Figure 3:** Diagram of the dynamics of the homeostatic stratified epithelium.

**Figure 4:** Diagram of viral dynamics when a HPV infection occurs.

**Figure 5:** Stability regions of infected equilibrium associated with the parameters (*σ*, *β*).

**Figure 6:** Dynamics of the model (18) when there is an infection generated by 100 virions with *σ* = 1000 and *β* = 9.447 × 10^−8^, such as *R*_0_ < 1.

**Figure 7:** Dynamics of the model (18) when there is an infection generated by 100 virions with *σ* = 1000 and *β* = 8.390 × 10^−4^, such as *R*_0_ > 1.

**Figure 8:** Dynamics of the model (18) when there is an infection generated by 100 virions with *σ* = 1000 and *β* = 7.247 × 10^−7^, such as *R*_0_ > 1.

**Figure 9:** Dynamics of the model (18) when there is an infection generated by 100 virions with *σ* = 1000 and *β* = 2.155 × 10^−6^, such as *R*_0_ > 1.

**Figure 10:** Dynamics of the model (18) when there is an infection generated by 100 virions with *σ* = 1000 and *β* = 1.447 × 10^−7^, such as *R*_0_ > 1.

**Figure 11:** Local sensitivity analysis of the basic reproduction number *R*_0_.

**Table 1:** Parameters of epithelial cellular dynamics of healthy tissue and dynamics of HPV infection.

Parameter	Description	Value	Unit	Ranges	Ref
*r*_*B*_	Uninfected stratum basale cell proliferation rate	0.07	day^−1^	[0.03; 0.07]	[25]
*r*_*B*_^∗^	Infected stratum basale cell proliferation rate	0.048	day^−1^	[−; −]	Fixed
*r*_*E*_	Uninfected stratum intermedium cell proliferation rate	0.039	day^−1^	[0.02; 1]	[25]
*r*_*E*_^∗^	Infected stratum intermedium cell proliferation rate	0.04	day^−1^	[−; −]	Fixed
*δ*_*B*_	Uninfected cell differentiation rate from stratum basale cell to stratum intermedium	0.044	day^−1^	[−; −]	[33]
*δ*_*B*_^∗^	Infected cell differentiation rate from stratum basale cell to stratum intermedium	0.05	day^−1^	[−; −]	Fixed
*δ*_*E*_	Uninfected cell differentiation rate from stratum intermedium cell to stratum corneum	0.099	day^−1^	[0.02; 1]	[25]
*δ*_*E*_^∗^	Infected cell differentiation rate from stratum intermedium cell to stratum corneum	0.118	day^−1^	[0; 5]	[25]
*μ*_*B*_	Uninfected basal cell natural death rate	0		[−; −]	[34]
*μ*_*B*_^∗^	Infected basal cell death rate	0		[−; −]	[34]
*μ*_*C*_	Desquamation rate of uninfected stratum corneum cells	0.27	day^−1^	[0.2; 1]	[25]
*μ*_*C*_^∗^	Desquamation rate of infected stratum corneum cells	0.27	day^−1^	[−; −]	Fixed
*K*_*B*_	Stratum basale cell carrying capacity	2693	cells	[1443; 13465]	[32]
*K*_*E*_	Stratum intermedium cell carrying capacity	2114	cells	[553; 5010]	[32]
*β*	Viral transmission rate	Varies	virion^−1^ · day^−1^	[10^−15^; 10^−5^]	[25]
*σ*	Production rate of free virions	Varies	cell^−1^ · virion · day^−1^	[10; 10^3^]	[11]
*γ*	Viral clearance rate	1.18	day^−1^	[0.2; 3]	[25]

[−; −] denotes ranges of values not evidenced in the literature.

## Data Availability

The data used to support the findings of this study are included within the article.
